# HIV/AIDS-Pneumonia Codynamics Model Analysis with Vaccination and Treatment

**DOI:** 10.1155/2022/3105734

**Published:** 2022-01-11

**Authors:** Shewafera Wondimagegnhu Teklu, Koya Purnachandra Rao

**Affiliations:** ^1^Department of Mathematics, Natural Science, Debre Berhan University, Debre Berhan, Ethiopia; ^2^Department O Mathematics, Natural Science, Wollega University, Nekemte, Ethiopia

## Abstract

In this paper, we proposed and analyzed a realistic compartmental mathematical model on the spread and control of HIV/AIDS-pneumonia coepidemic incorporating pneumonia vaccination and treatment for both infections at each infection stage in a population. The model exhibits six equilibriums: HIV/AIDS only disease-free, pneumonia only disease-free, HIV/AIDS-pneumonia coepidemic disease-free, HIV/AIDS only endemic, pneumonia only endemic, and HIV/AIDS-pneumonia coepidemic endemic equilibriums. The HIV/AIDS only submodel has a globally asymptotically stable disease-free equilibrium if *ℛ*_1_ < 1. Using center manifold theory, we have verified that both the pneumonia only submodel and the HIV/AIDS-pneumonia coepidemic model undergo backward bifurcations whenever *ℛ*_2_ < 1  and *ℛ*_3_ = max{*ℛ*_1_, *ℛ*_2_} < 1, respectively. Thus, for pneumonia infection and HIV/AIDS-pneumonia coinfection, the requirement of the basic reproduction numbers to be less than one, even though necessary, may not be sufficient to completely eliminate the disease. Our sensitivity analysis results demonstrate that the pneumonia disease transmission rate  *β*_2_ and the HIV/AIDS transmission rate  *β*_1_ play an important role to change the qualitative dynamics of HIV/AIDS and pneumonia coinfection. The pneumonia infection transmission rate *β*_2_ gives rises to the possibility of backward bifurcation for HIV/AIDS and pneumonia coinfection if *ℛ*_3_ = max{*ℛ*_1_, *ℛ*_2_} < 1, and hence, the existence of multiple endemic equilibria some of which are stable and others are unstable. Using standard data from different literatures, our results show that the complete HIV/AIDS and pneumonia coinfection model reproduction number is *ℛ*_3_ = max{*ℛ*_1_, *ℛ*_2_} = max{1.386, 9.69 } = 9.69  at *β*_1_ = 2 and *β*_2_ = 0.2  which shows that the disease spreads throughout the community. Finally, our numerical simulations show that pneumonia vaccination and treatment against disease have the effect of decreasing pneumonia and coepidemic disease expansion and reducing the progression rate of HIV infection to the AIDS stage.

## 1. Introduction

HIV/AIDS remains a major global health problem affecting approximately 70 million people worldwide causing significant morbidity and mortality (WHO, 2018) [1]. Over two-thirds of HIV/AIDS-infected population throughout the world is living in the sub-Saharan African Region [1–6]. AIDS is a common individual immune system disease caused by human immunodeficiency virus (HIV), i.e., RNA retrovirus which has developed into a global pandemic since the first patient was identified in 1981, making it one of the most destructive epidemics in history. HIV attacks human white blood cells and is transmitted through open sex, needle sharing, infected blood, and at childbirth [3, 6–9].

Pneumonia is one of the leading airborne infectious diseases caused by microorganisms such as bacteria, viruses, or fungi. It has been the common cause of morbidity and mortality in adults, children under five years of age, and HIV-mediated immunosuppression worldwide, and it is a treatable respiratory lung infectious disease [5, 10–14]. In most prospective microbiology-based studies, bacteria especially Streptococcus bacteria are identified in 30-50% of pneumonia cases which are a leading cause of pneumonia in developing countries [13, 15–17]. However, over the past, our understanding about transmission of pneumonia is basically based on research from high-income western countries but the WHO, 2018 report assessed that from 9.5 million annual death worldwide, pneumonia and other respiratory infections cause about 2 million child deaths yearly in developing countries [14, 18].

A coepidemic is the coexistence of two or more infections on a single individual at the population level [19]. HIV/AIDS-associated opportunistic infectious diseases are more common or more dangerous because of HIV immunosuppression [10].

Mathematical and statistical models of infectious diseases have, historically, provided useful insight into the transmission dynamics and control of infectious diseases [14]. Mathematical models have been used to investigate the dynamics of single infections and coepidemics, and HIV/AIDS-pneumonia is among the diseases that infect a large number of individuals worldwide [10, 17, 20, 21].

Babaei et al. [8] developed and analyzed a simple mathematical model for the interaction between drug addiction and the contagion of HIV/AIDS in Iranian prisons. They analyzed the stability of drug addiction and HIV/AIDS models separately with no medical treatment and investigated the impact of rehabilitating treatments on the control of HIV/AIDS spread in prisons, and finally, the reproduction numbers are compared in cases where there is no cure or some treatment methods are available. From their analysis, we have shown that their treatment methods for addiction withdrawal have a direct impact on the decrement and control of HIV/AIDS infection in prisons. Kizito et al. [13] constructed and discussed a mathematical model of treatment and vaccination impacts on pneumococcal pneumonia transmission dynamics. They found that, with treatment and vaccination combined, pneumonia can be eradicated; however, with treatment intervention alone, pneumonia remains in the population. Bakare and Nwozo [22] construct and analyzed a mathematical model for malaria–schistosomiasis coinfection. They have calculated the basic reproduction numbers and discussed the stability of equilibrium points of the model. They have shown the region where their model state variables become both mathematically and epidemiologically well-posed. They showed the model did not undergo backward bifurcation. Their mathematical modeling analysis result shows that intervention strategy suppresses the human-mosquito contact rate and human-snail contact rate to achieve malaria–schistosomiasis coepidemic free community. Shah et al. [3] formulated and analyzed a mathematical model for HIV/AIDS-TB coinfection considering HIV-infected population, and they found that medication plays a vital role in controlling the spread of the disease.

Limited mathematical modeling research analysis has been conducted on HIV/AIDS-pneumonia coepidemics, for prevention and controlling of the disease transmission with controlling and prevention mechanisms; however, theoretical sources such as [10, 15, 20, 21] show the coexistence of HIV/AIDS-pneumonia. For our new research article, we reviewed only two published HIV/AIDS-pneumonia coepidemic model articles. Nthiiri et al. [5] constructed mathematical modeling on HIV/AIDS-pneumonia coinfection with maximum protection against single HIV/AIDS, and pneumonia infections were their basic concern. They did not consider maximum protection against coinfection. In their model analysis, we have found that when protection is maximum, the number of HIV/AIDS and pneumonia cases is going down. Teklu and Mekonnen [6] constructed a deterministic mathematical model and analyzed it both mathematically and numerically. Our model considered treatment at each infection stage of the coinfection model, and we found that when the treatment rate increases, the number of infectious population at each infection stage decreases. Our model did not consider pneumonia vaccination.

We are motivated by the above studies especially the HIV/AIDS-pneumonia coexistence in the community; therefore, in this study, we considered the three center for disease control and prevention (CDC) stages of the HIV infection which are acute HIV infection, chronic HIV infection, and AIDS stage; we presented and analyzed a mathematical model describing the transmission dynamics of HIV/AIDS and pneumonia coinfection in a population where treatment for HIV/AIDS and both vaccination and treatment for pneumonia are available, respectively, in the community. Our model will be used to evaluate the effect of treatment at every infection stage of the HIV/AIDS only model, pneumonia only model, HIV/AIDS-pneumonia coinfection model, and effect of vaccination for pneumonia only model as control strategies for minimizing incidences of coinfections in the target population. The paper is organized as follows. The model is formulated in Section 2 and is analyzed in Section 3. Sensitivity analysis and numerical simulation were carried out in Section 4. Finally, discussion, conclusion, and recommendation of the study are carried out in Sections 5 and 6, respectively.

## 2. Mathematical Model Formulation

### 2.1. Assumptions and Descriptions

According to CDC the three HIV/AIDS infection stages, we divide the human population *N*(*t*) into twelve distinct classes as susceptible class to both HIV and pneumonia infections *Y*_1_(*t*), pneumonia vaccine class *Y*_2_ (*t*) , pneumonia-infected class *Y*_3_(*t*), acute HIV-infected class *Y*_4_(*t*), chronic HIV-infected class *Y*_5_(*t*), AIDS patient class *Y*_6_(*t*), acute HIV-pneumonia coepidemic class *Y*_7_(*t*), chronic HIV-pneumonia coepidemic class *Y*_8_(*t*), AIDS-pneumonia coepidemic class *Y*_9_(*t*), pneumonia treatment class *Y*_10_(*t*), HIV/AIDS treatment class *Y*_11_(*t*) entered from the three infection stages *Y*_4_(*t*), *Y*_5_(*t*), and *Y*_6_(*t*), and HIV/AIDS-pneumonia coepidemic treatment class *Y*_12_(*t*) entered from *Y*_7_(*t*), *Y*_8_(*t*), and *Y*_9_(*t*) cases such that

(1) $$\begin{array}{c} N\left(t\right)=Y_{1}\left(t\right)+Y_{2}\;\left(t\right)+Y_{3}\;\left(t\right)+Y_{4}\left(t\right)+Y_{5}\left(t\right)+Y_{6}\left(t\right)+Y_{7}\left(t\right)+Y_{8}\left(t\right)+Y_{9}\left(t\right)+Y_{10}\left(t\right)+Y_{11}\left(t\right)+Y_{12}\left(\text{t}\right). \end{array}$$

The susceptible class acquires HIV at the standard incidence rate given by

(2) $$\begin{array}{c} \lambda_{HC}\left(t\right)=\frac{\beta_{1}}{N}\left(Y_{4}\left(t\right)+\rho_{1}Y_{5}\left(t\right)+\rho_{2}Y_{7}\left(t\right)+\rho_{3}Y_{8}\left(t\right)\right), \end{array}$$

where *ρ*_3_ ≥ *ρ*_2_ ≥ *ρ*_1_ ≥ 1 is the modification rate that increases infectivity and *β*_1_ is the HIV/AIDS contagion rate.

The susceptible class acquires pneumonia at the mass action incidence rate

(3) $$\begin{array}{c} \lambda_{PC}\left(t\right)=\beta_{2}\left(Y_{3}\left(t\right)+\omega_{1}Y_{7}\left(t\right)+\omega_{2}Y_{8}\left(t\right)+\omega_{3}Y_{9}\left(t\right)\right), \end{array}$$

where *ω*_3_ > *ω*_2_ > *ω*_1_ is the modification rate that increases infectivity and *β*_2_ is the pneumonia contagion rate.

To construct the complete coepidemic dynamical system, we have assumed the following:

- A fraction of the population has been vaccinated before the disease outbreak at the portion of *π* and (1 − *π*) fraction of population entered to the vulnerable class
- The susceptible class is increased from the vaccinated class in which those individuals who are vaccinated but did not respond to vaccination with the waning rate of *τ* and from pneumonia-treated class in which those individuals who lose their temporary immunity by the rate *θ*
- Assume vaccination is not 100% effective, so vaccinated individuals also have a chance of being infected with proportion *ϵ*  of the serotype not covered by the vaccine where 0 ≤ *ϵ* < 1
- Individuals in a given compartment are homogeneous
- Assume no HIV transmission from *Y*_6_(*t*) and *Y*_9_(*t*) classes due to their reduced daily activities
- Individuals in each class are subject to natural mortality rate *d*
- The human population is variable
- We assumed there is no dual-infection transmission simultaneously
- Assume HIV has no vertical transmission and pneumonia is not naturally recovered
- No permanent immunity for pneumonia-infected individuals and become susceptible again after treatment

### 2.2. Schematic Diagram of the HIV/AIDS-Pneumonia Coepidemic Model

In this subsection using parameters in Table 1, variable definitions in Table 2, and the model assumptions and descriptions given in (2.1), the schematic diagram for the transmission of HIV/AIDS-pneumonia coepidemic is given by the diagram.

### 2.3. The HIV/AIDS-Pneumonia Coepidemic Dynamical System

From Figure 1, the HIV/AIDS and pneumonia coinfection dynamical system is given by

(4) $$\begin{array}{c} \begin{array}{c} \begin{array}{c} \begin{array}{c} \begin{array}{c} \begin{array}{c} \begin{array}{c} \frac{dY_{1}}{dt}=\left(1-\pi \right)\Lambda +\tau_{1}Y_{2}+\theta Y_{10}-\left(d+\lambda_{HC}+\lambda_{PC}\right)Y_{1},\\ \frac{dY_{2}}{dt}=\pi \Lambda -\epsilon \lambda_{PC}Y_{2}-\left(d+\tau_{1}+\lambda_{HC}\right)Y_{2}, \end{array}\\ \frac{dY_{3}}{dt}=\epsilon \lambda_{PC}Y_{2}+\lambda_{PC}Y_{1}-\left(\nu \lambda_{HC}+d+\kappa +d_{P}\right)Y_{3},\\ \frac{dY_{4}}{dt}=\lambda_{HC}Y_{1}+\lambda_{HC}Y_{2}-\left(d+\kappa_{1}+\delta_{1}+\psi_{1}\lambda_{PC}\right)Y_{4}, \end{array}\\ \frac{dY_{5}}{dt}=\delta_{1}Y_{4}-\left(d+\kappa_{2}+\delta_{2}+\psi_{2}\lambda_{PC}\right)Y_{5},\\ \frac{dY_{6}}{dt}=\delta_{2}H_{2}-\left(d+\kappa_{3}+d_{A}+\psi_{3}\lambda_{PC}\right)Y_{6}, \end{array}\\ \frac{dY_{7}}{dt}=\psi_{1}\lambda_{PC}Y_{4}+\nu \lambda_{H\text{C}}Y_{3}-\left(d+d_{P}+\sigma_{1}+\delta_{3}\right)Y_{7},\\ \frac{dY_{8}}{dt}=\psi_{2}\lambda_{PC}Y_{5}+\delta_{3}Y_{7}-\left(d+d_{P}+\sigma_{2}+\delta_{4}\right)Y_{8}, \end{array}\\ \frac{dY_{9}}{dt}=\psi_{3}\lambda_{PC}Y_{6}+\delta_{4}Y_{8}-\left(\text{d}+d_{AP}+\sigma_{3}\right)Y_{9},\\ \frac{dY_{10}}{dt}=\kappa Y_{3}-\left(d+\theta \right)Y_{10}, \end{array}\\ \frac{dY_{11}}{dt}=\kappa_{1}Y_{4}+\kappa_{2}Y_{5}+\kappa_{3}Y_{6}-dY_{11},\\ \frac{dY_{12}}{dt}=\sigma_{1}Y_{7}+\sigma_{2}Y_{8}+\sigma_{3}Y_{9}-dY_{12}. \end{array} \end{array}$$

With initial conditions,

(5) $$\begin{array}{c} \;Y_{1}\left(0\right)>0,\\ Y_{2}\left(0\right)\geq 0,\\ \;Y_{3}\left(0\right)\geq 0,\\ \;Y_{4}\left(0\right)\geq 0,\\ Y_{5}\left(0\right)\geq 0,\\ Y_{6}\left(0\right)\geq 0,\\ Y_{7}\left(0\right)\geq 0,\\ Y_{8}\left(0\right)\geq 0,\\ Y_{9}\left(0\right)\geq 0,\\ Y_{10}>0,\\ Y_{11}>0,\\ Y_{12}\left(0\right)\geq 0. \end{array}$$

The sum of all the differential equations in (4) is

(6) $$\begin{array}{c} \frac{dN}{dt}=\Lambda -dN-\left(d_{P}Y_{3}+d_{A}Y_{6}+d_{P}Y_{7}+d_{P}Y_{8}+d_{AP}Y_{9}\right), \end{array}$$

### 2.4. Positivity and Boundedness of the Solutions of the Model (4)

The model is mathematically analyzed by proving various theorems and algebraic computation dealing with different quantitative and qualitative attributes. Since the system deals with human populations which cannot be negative, we need to show that all the state variables are always nonnegative well as the solutions of system (4) remain positive with positive initial conditions (5) in the bounded region

(7) $$\begin{array}{c} \Omega =\left\{\left(Y_{1},Y_{2},Y_{3},Y_{4},Y_{5},Y_{6},Y_{7},Y_{8},Y_{9},Y_{10},Y_{11},Y_{12}\right)\in {\mathbb{R}}_{+}^{12},N\leq \frac{\Lambda }{d}\right\}. \end{array}$$

Here, in order for the model (4) to be epidemiologically well-posed, it is important to show that each state variable defined in Table 2 with positive initial conditions (5) is nonnegative for all time *t* > 0 in the bounded region given in (7).

**Theorem 1 .**

At the initial conditions (5), the solutions *Y*_1_(*t*), *Y*_2_(*t*), *Y*_3_(*t*), *Y*_4_(*t*), *Y*_5_(*t*),  *Y*_6_(*t*), *Y*_7_(*t*), *Y*_8_(*t*), *Y*_9_(*t*), *Y*_10_(*t*), *Y*_11_(*t*), and *Y*_12_(*t*) of system (4) are nonnegative for all time  *t* > 0.

**Proof**

Assume *Y*_1_(0) > 0, *Y*_2_(0) > 0, *Y*_3_(0) > 0, *Y*_4_(0) > 0, *Y*_5_(0) > 0, *Y*_6_(0) > 0, *Y*_7_(0) > 0, *Y*_8_(0) > 0, *Y*_9_(0) > 0, *Y*_10_(0) > 0, *Y*_11_(0), and *Y*_12_(0) > 0; then, for all *t* > 0, we have to prove that *Y*_1_ (*t*) > 0, *Y*_2_(*t*) > 0, *Y*_3_(*t*) > 0, *Y*_4_(*t*) > 0, *Y*_5_(*t*) > 0, *Y*_6_(*t*) > 0, *Y*_7_(*t*) > 0, *Y*_8_(*t*) > 0, *Y*_9_(*t*) > 0,  *Y*_10_(*t*) > 0, *Y*_11_(*t*) > 0, and *Y*_12_(*t*) > 0.

Define: *τ* = sup{*t* > 0 : *Y*_1_ (t) > 0, *Y*_2_(*t*) > 0, *Y*_3_(*t*) > 0,  *Y*_4_(*t*) > 0, *Y*_5_(*t*) > 0, *Y*_6_(*t*) > 0, *Y*_7_(*t*) > 0, *Y*_8_(*t*) > 0, *Y*_9_(*t*) > 0, *Y*_10_(*t*) > 0, *Y*_11_(*t*) > 0, and *Y*_12_(*t*) > 0}.

From the continuity of *Y*_1_(*t*), *Y*_2_(*t*), *Y*_3_(*t*), *Y*_4_(*t*),  *Y*_5_(*t*), *Y*_6_(*t*), *Y*_7_(*t*), *Y*_8_(*t*), *Y*_9_(*t*), *Y*_10_(*t*), *Y*_11_(*t*), and *Y*_12_(*t*)(*t*), we deduce that *τ* > 0. If *τ* = +∞, then positivity holds. But, if 0 < *τ* < +∞, *Y*_1_(*τ*) = 0 or *Y*_2_(*τ*) = 0 or *Y*_3_(*τ*) = 0 or *Y*_4_(*τ*) = 0 or *Y*_5_(*τ*) = 0 or *Y*_6_(*τ*) = 0 or *Y*_7_(*τ*) = 0 or *Y*_8_(*τ*) = 0 or *Y*_9_(*τ*) = 0 or *Y*_10_(*τ*) = 0 or *Y*_11_(*τ*) = 0 or *Y*_12_(0) = 0.

Here, from the first equation of the model (4), we have *dY*_1_/*dt* = (1 − *π*)*Λ* + *θY*_10_ + *τY*_2_ − (*d* + *λ*_*HC*_ + *λ*_*PC*_)*Y*_1._

Using the method of integrating factor, we obtained *Y*_1_(*τ*) = *M*_1_*Y*_1_(0) + *M*_1_∫_0_^*τ*^exp^∫(*d* + *λ*_*Hc*_(*t*) + *λ*_*Pc*_(*t*))*dt*^((1 − *π*)*Λ* + *θY*_10_(t) + *τY*_2_(*t*))*dt* > 0 where *M*_1_ = exp^−(*dτ* + ∫_0_^*τ*^(*λ*_*HC*_(*w*) + *λ*_*PC*_(*w*)*dw*)^ > 0, *Y*_1_(0) > 0, and from the definition of *τ*, we see that *Y*_2_(*t*) > 0,  *Y*_10_(*t*) > 0, and also the exponential function is always positive; then, the solution *Y*_1_(*τ*) > 0; hence, *Y*_1_(*τ*) ≠ 0. From the second equation of the model (4), we have *dY*_2_/*dt* = *πΛ* − (*d* + *τ*_1_ + *ϵλ*_*Pc*_ + *λ*_*Hc*_)*Y*_2_ and we have got *Y*_2_(*τ*) = *M*_1_*Y*_2_(0) + *M*_1_∫_0_^*τ*^exp^∫(*d* + *τ*_1_ + *ϵλ*_*Pc*_(*t*) + *λ*_*Hc*_(*t*))*dt*^(*πΛ*)*dt* > 0, where *M*_1_ = exp^−(*dτ* + *τ*_1_*τ* + ∫_0_^*τ*^(*λ*_*Hc*_(*w*) + *ϵλ*_*Pc*_(*w*)*dw*)^ > 0, *Y*_2_(0) > 0, and also, the exponential function always is positive; then, the solution *Y*_2_(*τ*) > 0; hence, *Y*_2_(*τ*) ≠ 0. Similarly, all the remaining state variables *Y*_3_(*τ*) > 0; hence, *Y*_3_(*τ*) ≠ 0 and *Y*_4_(*τ*) > 0; hence, *Y*_4_(*τ*) ≠ 0 and *Y*_5_(*τ*) > 0; hence, *Y*_5_(*τ*) ≠ 0 and *Y*_6_(*τ*) > 0; hence, *Y*_6_(*τ*) ≠ 0 and *Y*_7_(*τ*) > 0; hence, *Y*_7_(*τ*) ≠ 0 and *Y*_8_(*τ*) > 0; hence, *Y*_8_(*τ*) ≠ 0 and *Y*_9_(*τ*) > 0; hence, *Y*_9_(*τ*) ≠ 0 and *Y*_10_(*τ*) > 0; hence, *Y*_10_(*τ*) ≠ 0 and *Y*_11_(*τ*) > 0; hence, *Y*_11_(*τ*) ≠ 0 and *Y*_12_(*τ*) > 0; hence *Y*_12_(*τ*) ≠ 0. Thus, based on the definition of *τ*, it is not finite which means *τ* = +∞, and hence, all the solutions of system (2) are nonnegative.☐

**Theorem 2 .**

The region *Ω* given by (7) is bounded in ℝ_+_^12^.

**Proof**

Using equation (6), since all the state variables are nonnegative by Theorem 1, in the absence of infections, we have got *dN*/*dt* ≤ *Λ* − *dN*. By applying standard comparison theorem, we have got ∫(*dN*/(*Λ* − *dN*)) ≤ ∫*dt* and integrating both sides gives −(1/*d*)ln(*Λ* − *dN*) ≤ *t* + *c* where *c* is some constant, and after some steps of calculations, we have got 0 ≤ *N* (*t*) ≤ *Λ*/*d* which means all possible solutions of system (4) with positive initial conditions given in (5) enter in the bounded region (6).☐

## 3. The Mathematical Model Analysis

Before we analyze the HIV/AIDS-pneumonia coinfection model (4), we need to gain some background about the HIV/AIDS-only submodel and pneumonia-only submodel transmission dynamics.

### 3.1. HIV/AIDS Submodel Analysis

We have the HIV/AIDS submodel of (4) when *Y*_2_ = *Y*_3_ = *Y*_7_ = *Y*_8_ = *Y*_9_ = *Y*_10_ = *Y*_12_ = 0 which is given by

(8) $$\begin{array}{c} \begin{array}{c} \begin{array}{c} \frac{dY_{1}}{dt}=\Lambda -\left(d+\lambda_{H}\right)Y_{1},\\ \frac{dY_{4}}{dt}=\lambda_{H}Y_{1}-\left(d+\kappa_{1}+\delta_{1}\right)Y_{4},\\ \frac{dY_{5}}{dt}=\delta_{1}Y_{4}-\left(d+\kappa_{2}+\delta_{2}\right)Y_{5}, \end{array}\\ \frac{dY_{6}}{dt}=\delta_{2}Y_{5}-\left(d+\kappa_{3}+d_{A}\right)Y_{6},\\ \frac{dY_{11}}{dt}=\kappa_{1}Y_{4}+\kappa_{2}Y_{5}+\kappa_{3}Y_{6}-dY_{11}, \end{array} \end{array}$$

where the total population is *N*_1_(*t*) = *Y*_1_(*t*) + *Y*_4_(*t*) + *Y*_5_(*t*) + *Y*_6_(*t*) + *Y*_11_(*t*) and the HIV/AIDS single infection force of infection is given by *λ*_*H*_ = (*β*_1_/*N*_1_)(*Y*_4_ + *ρ*_1_*Y*_5_) with initial conditions *Y*_1_(0) > 0, *Y*_4_(0) ≥ 0, *Y*_5_(0) ≥ 0, *Y*_6_(0) ≥ 0, and *Y*_11_(0) ≥ 0.

Here, the detailed HIV/AIDS submodel model analysis is given in [6].

### 3.2. Pneumonia Submodel Analysis

From model (4), we have got the pneumonia submodel at *Y*_4_ = *Y*_5_ = *Y*_6_ = *Y*_7_= *Y*_8_=*Y*_9_ = *Y*_11_ = *Y*_12_ = 0, which is given by

(9) $$\begin{array}{c} \begin{array}{c} \begin{array}{c} \frac{dY_{1}}{dt}=\left(1-\pi \right)\Lambda +\tau_{1}Y_{2}+\theta Y_{10}-\left(d+\lambda_{P}\right)Y_{1},\\ \frac{dY_{2}}{dt}=\pi \Lambda -\epsilon \lambda_{P}Y_{2}-\left(d+\tau_{1}\right)Y_{2}, \end{array}\\ \frac{dY_{3}}{dt}=\epsilon \lambda_{P}Y_{2}+\lambda_{4}Y_{1}-\left(d+\kappa +d_{P}\right)Y_{3},\\ \frac{dY_{10}}{dt}=\kappa Y_{3}-\left(d+\theta \right)Y_{10}. \end{array} \end{array}$$

With initial conditions, *Y*_1_(0) > 0, *Y*_2_(0) ≥ 0, *Y*_3_(0) ≥ 0, *Y*_10_(0) ≥ 0, total population  *N*_2_(*t*) = *Y*_1_(*t*) + *Y*_2_(*t*) + *Y*_3_(*t*) + *Y*_10_(*t*), and pneumonia force of infection  *λ*_*P*_ = *β*_2_*Y*_3_(*t*).

In the region$\;\Omega_{2}=\left\{\begin{array}{c} \left(Y_{1},Y_{2},Y_{3},Y_{10}\right)\in {{\mathbb{R}}^{4}}_{+},N_{2}\leq \Lambda /d \end{array}\right\}$, it is easy to show that the set *Ω*_2_ is positively invariant and a global attractor of all positive solutions of submodel (9). Hence, it is sufficient to consider the dynamics of model (9) in *Ω*_2_ as epidemiologically and mathematically well-posed.

#### 3.2.1. Disease-Free Equilibrium Point of the Pneumonia Submodel

The disease-free equilibrium point of the pneumonia submodel is obtained by making the right-hand side of the system (15) as zero and setting the infectious class and treatment class to zero as *Y*_3_ = *Y*_10_ = 0 we have got

*Y*_1_^0^ = *Λ*(d + *τ*_1_) − *Λπ*d/*d*(d + *τ*_1_) and *Y*_2_^0^ = *Λπ*/(d + *τ*_1_) such that *E*_2_^0^ = (*Y*_1_^0^, *Y*_2_^0^, *Y*_3_^0^, *Y*_10_^0^) = ((*Λ*(d + *τ*_1_) − *Λπ*d/*d*(d + *τ*_1_)), (*Λπ*/d + *τ*_1_), 0, 0).

#### 3.2.2. The Effective Reproduction Number of the Pneumonia Submodel

The effective reproduction number measures the average number of new infections generated by a typically infectious individual in a community when some strategies are in place, like vaccination or treatment. We calculate the effective reproduction number  *ℛ*_2_ using the van den Driesch and Warmouth next-generation matrix approach [23]. The Effective reproduction number is the largest (dominant) eigenvalue (spectral radius) of the matrix *FV*^−1^ = [*∂ℱ*_*i*_(*E*_2_^0^)/*∂x*_*j*_][*∂ν*_*i*_(*E*_2_^0^)/*∂x*_*j*_]^−1^ where *ℱ*_*i*_ is the rate of appearance of new infection in compartment *i*, *ν*_*i*_ is the transfer of infections from one compartment *i* to another, and *E*_2_^0^ is the disease-free equilibrium point. Then, after a long calculation, we have got

(10) $$\begin{array}{c} F=\left[\begin{array}{cc} \frac{\beta_{2}\epsilon \Lambda \pi d+\beta_{2}\Lambda \left(\text{d}+\tau_{1}\right)-\beta_{2}\Lambda \pi \text{d}}{d\left(\text{d}+\tau_{1}\right)} & 0\\ 0 & 0 \end{array}\right],\\ \;V=\left[\begin{array}{cc} d+\kappa +d_{P} & 0\\ -\kappa & d+\theta \end{array}\right]. \end{array}$$

Then, using Mathematica, we have got

(11) $$\begin{array}{c} V^{-1}=\left[\begin{array}{cc} \frac{1}{d+\kappa +d_{P}} & 0\\ \frac{\gamma }{\left(\theta +d\right)\left(d+\kappa +d_{P}\right)} & \frac{1}{\theta +d} \end{array}\right],\\ FV^{-1}=\left[\begin{array}{cc} \frac{\beta_{2}\epsilon \Lambda \pi d+\beta_{2}\Lambda \left(\text{d}+\tau_{1}\right)-\beta_{2}\Lambda \pi \text{d}}{d\left(\text{d}+\tau_{1}\right)\left(d+\kappa +d_{P}\right)} & 0\\ 0 & 0 \end{array}\right]. \end{array}$$

The characteristic equation of the matrix *FV*^−1^ is

(12) $$\begin{array}{c} \left|\begin{array}{cc} \frac{\beta_{2}\epsilon \Lambda \pi d+\beta_{2}\Lambda \left(\text{d}+\tau_{1}\right)-\beta_{2}\Lambda \pi \text{d}}{d\left(\text{d}+\tau_{1}\right)\left(d+\kappa +d_{P}\right)}-\lambda & 0\\ 0 & 0-\lambda \end{array}\right|=0. \end{array}$$

Then, the spectral radius (effective reproduction number *ℛ*_2_) of *FV*^−1^ of the pneumonia submodel (9) is  *ℛ*_2_ = (*β*_2_*ϵΛπd* + *β*_2_*Λ*(d + *τ*_1_) − *β*_2_*Λπ*d)/(*d*(d + *τ*_1_)(*d* + *κ* + *d*_*P*_)). Here, *ℛ*_2_ is the effective reproduction number for pneumonia infection.

#### 3.2.3. Local and Global Stability of the Disease-Free Equilibrium Point

**Theorem 3 .**

The disease-free equilibrium point (DFE) *E*_2_^0^ of the pneumonia submodel (9) is locally asymptotically stable if *ℛ*_2_ < 1, otherwise unstable.

**Proof**

The local stability of the disease-free equilibrium of the system (9) can be studied from its Jacobian matrix at the disease-free equilibrium point *E*_2_^0^ = ((*Λ*(d + *τ*_1_) − *Λπ*d)/(*d*(d + *τ*_1_)), *Λπ*/(d + *τ*_1_ ), 0, 0) and Routh Hurwitz stability criteria. The Jacobian matrix of a dynamical system (9) at the disease-free equilibrium point is given by

(13) $$\begin{array}{c} J\left(E_{2}^{0}\right)=\left(\begin{array}{cccc} -d & \;\tau_{1} & \;\frac{-\beta_{2}\Lambda \left(\text{d}+\tau_{1}\right)+\beta_{2}\Lambda \pi \text{d}}{d\left(\text{d}+\tau_{1}\right)} & \theta \\ 0 & -\left(d+\tau_{1}\right) & \;\frac{-\epsilon \beta_{2}\Lambda \pi }{\text{d}+\tau_{1}} & 0\\ \;0 & 0 & \frac{\beta_{2}\epsilon \Lambda \pi d+\beta_{2}\Lambda \left(\text{d}+\tau_{1}\right)-\beta_{2}\Lambda \pi \text{d}}{d\left(\text{d}+\tau_{1}\right)}-\left(d+\kappa +d_{P}\right) & 0\\ 0 & 0 & \kappa & -\left(d+\theta \right) \end{array}\right). \end{array}$$

Then, the characteristic equation of the above Jacobian matrix is given by

(14) $$\begin{array}{c} \left|\begin{array}{cccc} -d-\lambda & \;\tau_{1} & \;\frac{-\beta_{2}\Lambda \left(\text{d}+\tau_{1}\right)+\beta_{2}\Lambda \pi \text{d}}{d\left(\text{d}+\tau_{1}\right)} & \theta \\ 0 & -\left(d+\tau_{1}\right)-\lambda & \;\frac{-\epsilon \beta_{2}\Lambda \pi }{\text{d}+\tau_{1}} & 0\\ \;0 & 0 & M-\lambda & 0\\ 0 & 0 & \kappa & -\left(d+\theta \right)-\lambda \end{array}\right|=0, \end{array}$$

where *M* = ((*β*_2_*ϵΛπd* + *β*_2_*Λ*(d + *τ*_1_) − *β*_2_*Λπ*d)/(*d*(*d* + *τ*_1_))) − (*d* + *κ* + *d*_*P*_).

After some steps, we have got *λ*_1_ = −*d* < 0 or *λ*_2_ = −(*d* + *τ*_1_) < 0 or *λ*_3_ = (*d* + *κ* + *d*_*P*_)[*ℛ*_2_ − 1] < 0 if *ℛ*_2_ < 1 or *λ*_4_ = −(*d* + *θ*) < 0. Therefore, since all the eigenvalues of the characteristics polynomial of the system (9) are negative if *ℛ*_2_ < 1, the disease-free equilibrium point of the pneumonia submodel is locally asymptotically stable.☐

#### 3.2.4. Existence of EEP for the Pneumonia Submodel

Let an arbitrary endemic equilibrium point of pneumonia-only dynamical system (9) be denoted by *E*_2_^∗^ = (*Y*_1_^∗^, *Y*_2_^∗^, *Y*_3_^∗^, *Y*_10_^∗^). Moreover, let *λ*_*P*_^∗^ = *β*_2_*Y*_3_^∗^ be the associated pneumonia mass action incidence rate (“force of infection”) at an equilibrium point. To find conditions for the existence of an arbitrary equilibrium point(s) for which pneumonia infection is endemic in the population, the equations of model (9) are solved in terms of the force of infection rate *λ*_*P*_^∗^ = *β*_2_*Y*_3_^∗^ at an endemic equilibrium point. Setting the right-hand sides of the equations of model (9) to zero and we have got *Y*_2_^∗^ = *πΛ*/(*ϵλ*_*P*_^∗^ + *d* + *τ*_1_), *Y*_10_^∗^ = *κY*_3_^∗^/(*d* + *θ*) and substitute *Y*_2_^∗^ and *Y*_10_^∗^  in to *Y*_1_^∗^, we obtain *Y*_1_^∗^ = ((1 − *π*)*Λ* + *τ*_1_*Y*_2_^∗^ + *θT*_*P*_^∗^)/(*d* + *λ*_*P*_^∗^) = ((1 − *π*)*Λ*/(*d* + *λ*_*P*_^∗^)*d* + *λ*_*P*_^∗^) + (*πΛτ*_1_/(*ϵλ*_*P*_^∗^ + *d* + *τ*_1_)(*d* + *λ*_*P*_^∗^)) + (*θγY*_3_^∗^/(*d* + *θ*)(*d* + *λ*_*P*_^∗^)) and substitute *Y*_2_^∗^ and *Y*_1_^∗^ in *Y*_3_^∗^, we obtain

(15) $$\begin{array}{c} Y_{3}^{*}=\frac{\pi \Lambda \epsilon \lambda_{P}^{*}\left(d+\kappa +d_{P}\right)\left(d+\theta \right)\left(d+\lambda_{P}^{*}\right)}{\left(d+\kappa +{\text{d}}_{P}\right)\left(\epsilon \lambda_{P}^{*}+d+\tau_{1}\right)\left[\left(d+\kappa +d_{P}\right)\left(d+\theta \right)\left(d+\lambda_{P}^{*}\right)-\theta \kappa \lambda_{P}^{*}\right]}+\frac{\left(1-\pi \right)\Lambda \lambda_{P}^{*}\left(d+\kappa +d_{P}\right)\left(d+\theta \right)\left(d+\lambda_{P}^{*}\right)}{\left(d+\kappa +d_{P}\right)\left(d+\lambda_{P}^{*}\right)\left[\left(d+\kappa +d_{P}\right)\left(d+\theta \right)\left(d+{\lambda_{P}}^{*}\right)-\theta \kappa \lambda_{P}^{*}\right]}+\frac{\pi \Lambda \tau_{1}\lambda_{P}^{*}\left(d+\kappa +d_{P}\right)\left(d+\theta \right)\left(d+\lambda_{P}^{*}\right)}{\left(d+\kappa +d_{P}\right)\left(\epsilon \lambda_{P}^{*}+d+\tau_{1}\right)\left(d+\lambda_{P}^{*}\right)\left[\left(d+\gamma +d_{P}\right)\left(d+\theta \right)\left(d+\lambda_{P}^{*}\right)-\theta \kappa \lambda_{P}^{*}\right]}. \end{array}$$

Finally, substitute *Y*_3_^∗^ in to pneumonia submodel (9) force of infection *λ*_*P*_^∗^ = *β*_2_*Y*_3_^∗^ as

(16) $$\begin{array}{c} \lambda_{P}^{*}=\beta_{2}Y_{3}^{*}=\frac{\beta_{2}\pi \Lambda \epsilon \lambda_{P}^{*}\left(d+\theta \right)\left(d+\lambda_{P}^{*}\right)}{\left(\epsilon \lambda_{P}^{*}+d+\tau_{1}\right)\left[\left(d+\kappa +d_{P}\right)\left(d+\theta \right)\left(d+\lambda_{P}^{*}\right)-\theta \kappa \lambda_{P}^{*}\right]}+\frac{\beta_{2}\left(1-\pi \right)\Lambda \lambda_{P}^{*}\left(d+\theta \right)}{\left[\left(d+\kappa +d_{P}\right)\left(d+\theta \right)\left(d+\lambda_{P}^{*}\right)-\theta \kappa \lambda_{P}^{*}\right]}+\frac{\beta_{2}\pi \Lambda \tau_{1}\lambda_{P}^{*}\left(d+\theta \right)}{\left(\epsilon \lambda_{P}^{*}+\kappa +\tau_{1}\right)\left[\left(d+\kappa +d_{P}\right)\left(d+\theta \right)\left(d+\lambda_{P}^{*}\right)-\theta \kappa \lambda_{P}^{*}\right]}, \end{array}$$

and letting *m*_1_ = *d* + *κ* + *d*_*P*_, *m*_2_ = *d* + *τ*_1_, and *m*_3_ = *d* + *θ*, we have got *a*_2_*λ*_*P*_^∗^^2^+*a*_1_*λ*_*P*_^∗^+*a*_0_ = 0 where *a*_2_ = *m*_1_*m*_3_*ϵ* − *θκϵ* > 0,  *a*_1_ = *m*_1_*m*_3_*dϵ* + *m*_1_*m*_2_*m*_3_ − *m*_2_*θκ* − *β*_2_*Λm*_3_*ϵ*, and *a*_0_ = *m*_1_*m*_2_*m*_3_*μ*[1 − *ℛ*_2_] > 0 if *ℛ*_2_ < 1.

Here, the nonzero equilibrium(s) of the model (9) satisfies *f*(*λ*_*P*_^∗^) = *a*_2_*λ*_*P*_^∗^^2^ + *a*_1_*λ*_*P*_^∗^ + *a*_0_ = 0 so that the quadratic equation can be analyzed for the possibility of multiple equilibriums. It is worth noting that the coefficient *a*_2_ is always positive and *a*_0_ is positive (negative) if *ℛ*_*P*_ is less than (greater than) unity, respectively. Hence, we have established the following result.

**Theorem 4 .**

The pneumonia submodel (9) has the following:

- Exactly one unique endemic equilibrium if *a*_0_ < 0 (i.e., *ℛ*_2_>1)
- Exactly one unique endemic equilibrium if *a*_1_<0, and *a*_0_ = 0 or *a*_1_^2^ − 4*a*_2_*a*_0_ = 0
- Exactly two endemic equilibriums if *a*_0_ > 0 (i.e., *ℛ*_2_ < 1), *a*_1_ < 0, and *a*_1_^2^ − 4*a*_2_*a*_0_ > 0
- No endemic equilibrium otherwise

Here, item (iii) shows the happening of the backward bifurcation in pneumonia submodel (9), i.e., the locally asymptotically stable disease-free equilibrium point coexists with a locally asymptotically stable endemic equilibrium point if *ℛ*_2_ < 1; examples of the existence of backward bifurcation phenomenon in mathematical epidemiological models, and the causes, can be seen in [2, 9, 22, 24–26]. The epidemiological consequence is that the classical epidemiological requirement of having the reproduction number *ℛ*_2_ to be less than one, even though necessary, is not sufficient for the effective control of the disease. The existence of the backward bifurcation phenomenon in submodel (9) is now explored.

#### 3.2.5. Bifurcation Analysis

It is instructive to explore the possibility of backward bifurcation in model (9).

**Theorem 5 .**

Model (9) exhibits backward bifurcation at *ℛ*_2_ = 1 whenever the inequality *D*_1_ > *D*_2_ holds.

Here, we apply the center manifold theory in [27]; however, to apply this theory, the following simplification and change of variables are made.

Let *Y*_1_ = *x*_1_,*Y*_2_ = *x*_2_, *Y*_3_ = *x*_3_, and *Y*_10_ = *x*_4_ such that *N*_2_ = *x*_1_ + *x*_2_ + *x*_3_ + *x*_4_. Furthermore, by using vector notation *X* = (*x*_1_, *x*_2_, *x*_3_, *x*_4_)^*T*^, pneumonia submodel (9) can be written in the form *dX*/*dt* = *F*(*X*) with

*F* = (*f*_1_, *f*_2_, *f*_3_, *f*_4_)^*T*^, as follows:

(17) $$\begin{array}{c} \begin{array}{c} \begin{array}{c} \frac{{dx}_{1}}{dt}=f_{1}=\left(1-\pi \right)\Lambda +\tau_{1}x_{2}+\theta x_{4}-\left(d+\lambda_{P}\right)x_{1},\\ \frac{{dx}_{2}}{dt}=f_{2}=\pi \Lambda -\left(\epsilon \lambda_{P}+d+\tau_{1}\right)x_{2}, \end{array}\\ \frac{{dx}_{3}}{dt}=f_{3}=\epsilon \lambda_{P}x_{2}+\lambda_{P}x_{1}-\left(d+\kappa +d_{P}\right)x_{3},\\ \frac{{dx}_{4}}{dt}=f_{4}=\kappa x_{3}-\left(d+\theta \right)x_{4}, \end{array} \end{array}$$

with *λ*_*P*_ = *β*_2_*x*_3_, then the method entails evaluating the Jacobian of system (17) at the DFE point *E*_2_^0^, denoted by *J*(*E*_2_^0^), and this gives us

(18) $$\begin{array}{c} J\left(E_{2}^{0}\right)=\left(\begin{array}{cccc} -d & \;\tau_{1} & \;\frac{-\beta_{2}\Lambda \left(d+\tau_{1}\right)+\beta_{2}\Lambda \pi d}{d\left(d+\tau_{1}\right)} & \theta \\ 0 & -\left(d+\tau_{1}\right) & \;\frac{-\epsilon \beta_{2}\Lambda \pi }{\mu +\tau_{1}} & 0\\ \;0 & 0 & \frac{\beta_{2}\epsilon \Lambda \pi d+\beta_{2}\Lambda \left(d+\tau_{1}\right)-\beta_{2}\Lambda \pi \mu }{d\left(d+\tau_{1}\right)}-\left(d+\kappa +d_{P}\right) & 0\\ 0 & 0 & \kappa & -\left(d+\theta \right) \end{array}\right). \end{array}$$

Consider, next, the case when *ℛ*_*P*_ = 1. Suppose, further, that *β*_2_ = *β*^∗^  is chosen as a bifurcation parameter.

Solving for *β*_2_ from *ℛ*_2_ = 1 as *ℛ*_2_ = *β*_2_*ϵΛπd* + *β*_2_*Λ*(*d* + *τ*_1_) − *β*_2_*Λπd*/*d*(*d* + *τ*_1_)(*d* + *κ* + *d*_*P*_) = 1 and we have got *β*_2_ = *β*^∗^ = *d*(d + *τ*_1_)(*d* + *κ* + *d*_*P*_)/*ϵΛπd* + *Λ*(d + *τ*_1_) − *Λπ*d and

(19) $$\begin{array}{c} J_{\beta^{*}}=\left(\begin{array}{cccc} -d & \;\tau_{1} & \;\frac{-\beta^{*}\Lambda \left(\text{d}+\tau_{1}\right)+\beta^{*}\Lambda \pi \text{d}}{d\left(\text{d}+\tau_{1}\right)} & \theta \\ 0 & -\left(d+\tau_{1}\right) & \;\frac{-\epsilon \beta^{*}\Lambda \pi }{\text{d}+\tau_{1}} & 0\\ \;0 & 0 & \frac{\beta^{*}\epsilon \Lambda \pi d+\beta^{*}\Lambda \left(\text{d}+\tau_{1}\right)-\beta^{*}\Lambda \pi \text{d}}{d\left(\text{d}+\tau_{1}\right)}-\left(d+\kappa +d_{P}\right) & 0\\ 0 & 0 & \gamma & -\left(\mu +\theta \right) \end{array}\right). \end{array}$$

After some steps of the calculation, we have got the eigenvalues of *J*_*β*^∗^_ as *λ*_1_ = −*d* or *λ*_2_ = −(*d* + *τ*_1_) or *λ*_3_ = 0 or *λ*_4_ = −(*d* + *θ*).

It follows that the Jacobian *J*(*E*_2_^0^) of (17) at the DFE, with *β*_2_ = *β*^∗^, denoted by *J*_*β*^∗^_, has a simple zero eigenvalue with all the remaining eigenvalues having a negative real part. Hence, the center manifold theory [27] can be used to analyze the dynamics of model (9). In particular, Theorem 2 of Castillo-Chavez and Song [28] will be used to show that model (9) undergoes backward bifurcation at *ℛ*_2_ = 1

Eigenvectors of *J*_*β*^∗^_: for the case *ℛ*_2_ = 1, it can be shown that the Jacobian of (29) at *β*_2_ = *β*^∗^ (denoted by *J*_*β*^∗^_) has a right eigenvectors associated with the zero eigenvalue given by *u* = (*u*_1_, *u*_2_, *u*_3_, *u*_4_)^*T*^ with values

(20) $$\begin{array}{c} u_{1}=\left[\frac{-\epsilon \beta^{*}\Lambda \pi d\tau_{1}\left(d+\theta \right)-\beta^{*}\Lambda {\left(\text{d}+\tau_{1}\right)}^{2}\left(d+\theta \right)+\beta^{*}\Lambda \pi \text{d}\left(\text{d}+\tau_{1}\right)\left(d+\theta \right)+\theta \kappa d{\left(\text{d}+\tau_{1}\right)}^{2}}{d^{2}{\left(\text{d}+\tau_{1}\right)}^{2}}\right]\;u_{3},\\ \;u_{2}=-\frac{\epsilon \beta^{*}\Lambda \pi }{{\left(\text{d}+\tau_{1}\right)}^{2}}u_{3},\\ u_{3}=u_{3}>0,\\ u_{4}=\frac{\kappa }{d+\theta }u_{3}. \end{array}$$

Similarly, the left eigenvector associated with the zero eigenvalues at *β*_2_ = *β*^∗^ given by *v* = (*v*_1_, *v*_2_, *v*_3_, *v*_4_)^*T*^ are *v*_1_ = *v*_2_ = *v*_4_ = 0, *v*_3_ = *v*_3_ > 0.

After long calculations, the bifurcation coefficients *a* and *b* are obtained as *a* = *D*_1_ − *D*_2_ where *D*_1_=*β*^∗^*Λπd*(*d* + *τ*_1_)(*d* + *θ*) + *θκd*(*d* + *τ*_1_)^2^/*d*^2^(*d* + *τ*_1_)^2^, and  *D*_2_ = (*ϵβ*^∗^*Λπdτ*_1_(*d* + *θ*) + *β*^∗^*Λ*(*d* + *τ*_1_)^2^(*d* + *θ*)/*d*^2^(*d* + *τ*_1_)^2^) + *ϵ*(*ϵβ*^∗^*Λπ*/(d + *τ*_1_)^2^).

Thus, the bifurcation coefficient *a* is positive if *D*_1_ > *D*_2_. Furthermore,  *b* = *v*_3_*u*_2_*u*_3_(*Λ*(*d* + *τ*_1_) − *Λπd*/*d*(*d* + *τ*_1_)) > 0.

Hence, from in Castillo-Chavez and Song [28], model (9) exhibits a backward bifurcation at *ℛ*_2_ = 1 whenever *D*_1_ > *D*_2_.

### 3.3. Analysis of the Full HIV/AIDS-Pneumonia Coinfection

Having analyzed the dynamics of the two submodels, that is, HIV/AIDS submodel (8) and the pneumonia submodel (9), the complete HIV/AIDS-pneumonia coinfection model (4) is now considered (the analysis is done in the positively invariant region *Ω* given in (7)).

#### 3.3.1. Disease-Free Equilibrium Point of the HIV/AIDS-Pneumonia Coinfection

The disease-free equilibrium point of model (4) is obtained by setting all the infectious classes and treatment classes to zero such that  *Y*_3_ = *Y*_4_ = *Y*_5_ = *Y*_6_ = *Y*_7_ = *Y*_8_ = *Y*_9_ = *Y*_10_ = *Y*_11_ = *Y*_12_ = 0 and hence *E*_3_^0^== (*Λ*(*d* + *τ*_1_) − *Λπd*/*d*(*d* + *τ*_1_), *Λπ*/(*d* + *τ*_1_ ), 0, 0, 0, 0, 0, 0, 0, 0, 0, 0).

#### 3.3.2. Effective Reproduction Number of the HIV/AIDS-Pneumonia Coinfection

The basic reproduction number, denoted by *ℛ*_0_, is the expected number of secondary cases produced, in a completely susceptible population, by a typical infective individual [6, 23, 28]. For simple classical models if *ℛ*_0_ < 1, then it means that on average, an infected individual infects less than one susceptible over the course of its infectious period and the disease cannot grow. If however, *ℛ*_0_ > 1, then an infected individual infects more than one susceptible over the course of its infectious period and the disease will persist. For more complicated models with several infected compartments, this simple heuristic definition of *ℛ*_0_ is insufficient [23]. Due to its importance, researchers have sought to find ways of determining *ℛ*_0_. Two important concepts in modeling outbreaks of infectious diseases are the basic reproduction number, universally denoted by *ℛ*_0_ and the generation time (the average time from symptom onset in a primary case to symptom onset in a secondary case), which jointly determine the likelihood and speed of epidemic outbreaks [29].

Here, we calculated the HIV/AIDS-pneumonia coinfection effective reproduction number *ℛ*_3_ of model (4) using the van den Driesch and Warmouth next-generation matrix approach [23]. The effective reproduction number is the largest (dominant) eigenvalue (spectral radius) of the matrix *FV*^−1^ = [*∂ℱ*_*i*_(*E*_3_^0^)/*∂x*_*j*_][*∂ν*_*i*_(*E*_3_^0^)/*∂x*_*j*_]^−1^ where *ℱ*_*i*_ is the rate of appearance of new infection in compartment *i* , *ν*_*i*_ is the transfer of infections from one compartment *i* to another, and *E*_3_^0^ is the disease-free equilibrium point *E*_3_^0^ = (*Λ*(d + *τ*_1_) − *Λπ*d/*d*(d + *τ*_1_), *Λπ*/d + *τ*_1_, 0, 0, 0, 0, 0, 0, 0, 0, 0, 0).

After long detailed calculations, the transition matrix *F* is given by

(21) $$\begin{array}{c} \text{F}=\left[\begin{array}{cccccccccc} A & 0 & 0 & 0 & 0 & 0 & 0 & 0 & 0 & 0\\ 0 & \beta_{1} & \beta_{1}\rho_{1} & 0 & 0 & 0 & 0 & 0 & 0 & 0\\ 0 & 0 & 0 & 0 & 0 & 0 & 0 & 0 & 0 & 0\\ 0 & 0 & 0 & 0 & 0 & 0 & 0 & 0 & 0 & 0\\ 0 & 0 & 0 & 0 & 0 & 0 & 0 & 0 & 0 & 0\\ 0 & 0 & 0 & 0 & 0 & 0 & 0 & 0 & 0 & 0\\ 0 & 0 & 0 & 0 & 0 & 0 & 0 & 0 & 0 & 0\\ 0 & 0 & 0 & 0 & 0 & 0 & 0 & 0 & 0 & 0\\ 0 & 0 & 0 & 0 & 0 & 0 & 0 & 0 & 0 & 0\\ 0 & 0 & 0 & 0 & 0 & 0 & 0 & 0 & 0 & 0 \end{array}\right], \end{array}$$

and the transmission matrix *V* is given by

(22) $$\begin{array}{c} V=\left[\begin{array}{cccccccccc} D_{1} & 0 & 0 & 0 & 0 & 0 & 0 & 0 & 0 & 0\\ 0 & D_{2} & 0 & 0 & 0 & 0 & 0 & 0 & 0 & 0\\ 0 & -\delta_{1} & D_{3} & 0 & 0 & 0 & 0 & 0 & 0 & 0\\ 0 & 0 & -\delta_{2} & D_{4} & 0 & 0 & 0 & 0 & 0 & 0\\ 0 & 0 & 0 & 0 & D_{5} & 0 & 0 & 0 & 0 & 0\\ 0 & 0 & 0 & 0 & -\delta_{3} & D_{6} & 0 & 0 & 0 & 0\\ 0 & 0 & 0 & 0 & 0 & -\delta_{4} & D_{7} & 0 & 0 & 0\\ -\kappa & 0 & 0 & 0 & 0 & 0 & 0 & \theta & 0 & 0\\ 0 & -\kappa_{1} & -\kappa_{2} & -\kappa_{3} & 0 & 0 & 0 & 0 & d & 0\\ 0 & 0 & 0 & 0 & -\sigma_{1} & -\sigma_{2} & -\sigma_{3} & 0 & 0 & d \end{array}\right], \end{array}$$

where *D*_1_ = *d* + *κ* + *d*_*P*_, *D*_2_ = *d* + *κ*_1_ + *δ*_1_, *D*_3_ = *d* + *κ*_2_ + *δ*_2_, *D*_4_ = *d* + *κ*_3_ + *d*_*A*_, *D*_5_ = *d* + *d*_*P*_ + *σ*_1_ + *δ*_3_, *D*_6_ = *d* + *d*_*P*_ + *σ*_2_ + *δ*_4_, and *D*_7_ = *d* + *d*_*AP*_ + *ε*_3_.

Then, by using Mathematica, we have got

(23) $$\begin{array}{c} FV^{-1}=\left[\begin{array}{cccccccccc} \frac{\left(\pi \epsilon \Lambda \beta_{2}/d+\tau_{1}\right)+\beta_{2}\left[-\pi \Lambda d+\Lambda \left[d+\tau_{1}\right]/d\left[d+\tau_{1}\right]\right]}{D_{1}} & 0 & 0 & 0 & 0 & 0 & 0 & 0 & 0 & 0\\ 0 & \frac{\beta_{1}}{D_{2}}+\frac{\delta_{1}\beta_{1}\rho_{1}}{D_{2}D_{3}} & \frac{\beta_{1}\rho_{1}}{D_{3}} & 0 & 0 & 0 & 0 & 0 & 0 & 0\\ 0 & 0 & 0 & 0 & 0 & 0 & 0 & 0 & 0 & 0\\ 0 & 0 & 0 & 0 & 0 & 0 & 0 & 0 & 0 & 0\\ 0 & 0 & 0 & 0 & 0 & 0 & 0 & 0 & 0 & 0\\ 0 & 0 & 0 & 0 & 0 & 0 & 0 & 0 & 0 & 0\\ 0 & 0 & 0 & 0 & 0 & 0 & 0 & 0 & 0 & 0\\ 0 & 0 & 0 & 0 & 0 & 0 & 0 & 0 & 0 & 0\\ 0 & 0 & 0 & 0 & 0 & 0 & 0 & 0 & 0 & 0\\ 0 & 0 & 0 & 0 & 0 & 0 & 0 & 0 & 0 & 0 \end{array}\right]. \end{array}$$

The characteristic equation of the matrix *FV*^−1^ is given by

(24) $$\begin{array}{c} \left|\begin{array}{cccccccccc} \left(A_{1}-\lambda \right) & 0 & 0 & 0 & 0 & 0 & 0 & 0 & 0 & 0\\ 0 & \left(B-\lambda \right) & \frac{\beta_{1}\rho_{1}}{D_{3}} & 0 & 0 & 0 & 0 & 0 & 0 & 0\\ 0 & 0 & \left(0-\lambda \right) & 0 & 0 & 0 & 0 & 0 & 0 & 0\\ 0 & 0 & 0 & \left(0-\lambda \right) & 0 & 0 & 0 & 0 & 0 & 0\\ 0 & 0 & 0 & 0 & \left(0-\lambda \right) & 0 & 0 & 0 & 0 & 0\\ 0 & 0 & 0 & 0 & 0 & \left(0-\lambda \right) & 0 & 0 & 0 & 0\\ 0 & 0 & 0 & 0 & 0 & 0 & \left(0-\lambda \right) & 0 & 0 & 0\\ 0 & 0 & 0 & 0 & 0 & 0 & 0 & \left(0-\lambda \right) & 0 & 0\\ 0 & 0 & 0 & 0 & 0 & 0 & 0 & 0 & \left(0-\lambda \right) & 0\\ 0 & 0 & 0 & 0 & 0 & 0 & 0 & 0 & 0 & \left(0-\lambda \right) \end{array}\right|=0, \end{array}$$

where *A*_1_ = (*πϵΛβ*_2_/(*d* + *τ*_1_)) + *β*_2_[(−*πΛd* + *Λ*[*d* + *τ*_1_]/*d*[*d* + *τ*_1_])]/*D*_1_, *B* = (*β*_1_/*D*_2_) + (*δ*_1_*β*_1_*ρ*_1_/*D*_2_*D*_3_);  then, the eigenvalues of *FV*^−1^ are *λ*_1_ = *β*_2_*ϵπdΛ* + *β*_2_*Λ*[*d* + *τ*_1_] − *β*_2_*πΛd*/*D*_1_(*d* + *τ*_1_) or *λ*_2_ = (*β*_1_/*D*_2_) + *δ*_1_*β*_1_*ρ*_1_/*D*_2_*D*_3_  or *λ*_3_ = *λ*_4_ = *λ*_5_ = *λ*_6_ = *λ*_7_ = *λ*_8_ = *λ*_9_ = *λ*_10_ = 0.

Thus, the effective reproduction number of the HIV/AIDS-pneumonia coinfection dynamical system (4) is the dominant eigenvalue of the matrix *FV*^−1^ which is given by

*ℛ*_3_ = max{*λ*_1_, *λ*_2_} = max{*β*_2_*ϵπdΛ* + *β*_2_*Λ*[*d* + *τ*_1_] − *β*_2_*πΛd*/*D*_1_(*d* + *τ*_1_), (*β*_1_/*D*_2_) + (*δ*_1_*β*_1_*ρ*_1_/*D*_2_*D*_3_)}. Here,  *ℛ*_2_ = *β*_2_*ϵπdΛ* + *β*_2_*Λ*[*d* + *τ*_1_] − *β*_2_*πΛd*/(*d* + *κ* + *d*_*P*_)(*d* + *τ*_1_) is the effective reproduction number for pneumonia-only infected individual and *ℛ*_1_ = (*β*_1_/(*d* + *κ*_1_ + *δ*_1_)) + (*β*_1_*ρ*_1_*δ*_1_/(*d* + *κ*_1_ + *δ*_1_)(*d* + *κ*_2_ + *κ*_2_)) is the basic reproduction for HIV/AIDS-only infected individual.

Here, *ℛ*_1_ represent the basic reproduction number for HIV/AIDS submodel,  *ℛ*_2_ and *ℛ*_3_ are the effective reproduction numbers for the pneumonia submodel and HIV/AIDS-pneumonia coinfection model, respectively. The following three outcomes are possible: (i) for *ℛ*_1_ < 1, the HIV/AIDS submodel disease-free steady state *E*_1_ is globally stable in the region *Ω*_1_, and HIV is not spreading in the community; (ii) for *ℛ*_2_ < 1, then *E*_2_ is not globally stable in the region *Ω*_2_, and pneumonia may spread through the community; (iii) for *ℛ*_3_ < 1, the steady state *E*_3_ is not globally stable in the region *Ω*, and HIV/AIDS-pneumonia coinfection may spread through the community.

Note that none of the parameters corresponding to coinfection treatment (i.e., *σ*_1_ or *σ*_2_ or *σ*_3_) are present in the expression for *ℛ*_3_, indicating no impact of treating coinfected population on *ℛ*_3_.

#### 3.3.3. Locally Asymptotically Stability of the Disease-Free Equilibrium (DFE)

**Theorem 6 .**

The disease-free equilibrium of model (4) above is locally asymptotically stable if *ℛ*_3_ < 1, otherwise unstable.

**Proof**

The Jacobian matrix *J*(*E*_3_^0^) of model (4) at *E*_3_^0^ is given by

(25) $$\begin{array}{c} J\;\left(E_{3}^{0}\right)=\left[\begin{array}{cccccccccccc} -d & \tau_{1} & -\beta_{2}Y_{1}^{0} & -\frac{\beta_{1}}{N^{0}}Y_{1}^{0} & -\frac{\beta_{1}}{N^{0}}\rho_{1}Y_{1}^{0} & 0 & 0 & 0 & \theta & 0 & 0 & 0\\ 0 & -d-\tau_{1} & -\beta_{2}\epsilon Y_{2}^{0} & -\frac{\beta_{1}}{N^{0}}Y_{2}^{0} & -\frac{\beta_{1}}{N^{0}}\rho_{1}Y_{2}^{0} & 0 & 0 & 0 & 0 & 0 & 0 & 0\\ 0 & 0 & Z_{1} & 0 & 0 & 0 & 0 & 0 & 0 & 0 & 0 & 0\\ 0 & 0 & 0 & Z_{2} & \frac{\beta_{1}}{N^{0}}\rho_{1}Y_{1}^{0} & 0 & 0 & 0 & 0 & 0 & 0 & 0\\ 0 & 0 & 0 & \delta_{1} & Z_{3} & 0 & 0 & 0 & 0 & 0 & 0 & 0\\ 0 & 0 & 0 & 0 & \delta_{2} & Z_{4} & 0 & 0 & 0 & 0 & 0 & 0\\ 0 & 0 & 0 & 0 & 0 & 0 & Z_{5} & 0 & 0 & 0 & 0 & 0\\ 0 & 0 & 0 & 0 & 0 & 0 & \delta_{3} & Z_{6} & 0 & 0 & 0 & 0\\ 0 & 0 & 0 & 0 & 0 & 0 & 0 & \delta_{4} & Z_{7} & 0 & 0 & 0\\ 0 & 0 & \kappa & 0 & 0 & 0 & 0 & 0 & 0 & Z_{8} & 0 & 0\\ 0 & 0 & 0 & \kappa_{1} & \kappa_{2} & \kappa_{3} & 0 & 0 & 0 & 0 & -d & 0\\ 0 & 0 & 0 & 0 & 0 & 0 & \sigma_{1} & \sigma_{2} & \sigma_{3} & 0 & 0 & -d \end{array}\right], \end{array}$$

where *Z*_1_ = *β*_2_*ϵY*_2_^0^ + *β*_2_*Y*_1_^0^ − (*d* + *κ* + *d*_*P*_), *Z*_2_ = (*β*_1_/*N*^0^)*Y*_1_^0^ − (*d* + *κ*_1_ + *δ*_1_),  *Z*_3_ = −(*d* + *κ*_2_ + *δ*_2_),  *Z*_4_ = −(*d* + *κ*_3_ + *d*_*A*_), *Z*_5_ = −(*d* + *d*_*P*_ + *σ*_1_ + *δ*_3_), *Z*_6_ = −(*d* + *d*_*P*_ + *σ*_2_ + *δ*_4_), *Z*_7_ = −(*d* + *d*_*AP*_ + *σ*_3_), and *Z*_8_ = −(*d* + *θ*).

Then, the characteristic equation of the Jacobian matrix *J* (*E*_3_^0^) is given by

(26) $$\begin{array}{c} \left|\begin{array}{cccccccccccc} -d-\lambda & \tau_{1} & -\beta_{2}Y_{1}^{0} & -\frac{\beta_{1}}{N^{0}}Y_{1}^{0} & -\frac{\beta_{1}}{N^{0}}\rho_{1}Y_{1}^{0} & 0 & 0 & 0 & 0 & \theta & 0 & 0\\ 0 & -d-\tau_{1}-\lambda & -\beta_{2}\epsilon Y_{2}^{0} & -\frac{\beta_{1}}{N^{0}}Y_{2}^{0} & -\frac{\beta_{1}}{N^{0}}\rho_{1}Y_{2}^{0} & 0 & 0 & 0 & 0 & 0 & 0 & 0\\ 0 & 0 & Z_{1}-\lambda & 0 & 0 & 0 & 0 & 0 & 0 & 0 & 0 & 0\\ 0 & 0 & 0 & Z_{2}-\lambda & \frac{\beta_{1}}{N^{0}}\rho_{1}Y_{1}^{0} & 0 & 0 & 0 & 0 & 0 & 0 & 0\\ 0 & 0 & 0 & \delta_{1} & Z_{3}-\lambda & 0 & 0 & 0 & 0 & 0 & 0 & 0\\ 0 & 0 & 0 & 0 & \delta_{2} & Z_{4}-\lambda & 0 & 0 & 0 & 0 & 0 & 0\\ 0 & 0 & 0 & 0 & 0 & 0 & Z_{5}-\lambda & 0 & 0 & 0 & 0 & 0\\ 0 & 0 & 0 & 0 & 0 & 0 & \delta_{3} & Z_{6}-\lambda & 0 & 0 & 0 & 0\\ 0 & 0 & 0 & 0 & 0 & 0 & 0 & \delta_{4} & Z_{7}-\lambda & 0 & 0 & 0\\ 0 & 0 & \kappa & 0 & 0 & 0 & 0 & 0 & 0 & Z_{8}-\lambda & 0 & 0\\ 0 & 0 & 0 & \kappa_{1} & \kappa_{2} & \kappa_{3} & 0 & 0 & 0 & 0 & -d-\lambda & 0\\ 0 & 0 & 0 & 0 & 0 & 0 & \sigma_{1} & \sigma_{2} & \sigma_{3} & 0 & 0 & -d-\lambda \end{array}\right|=0. \end{array}$$

After detailed calculations, we have got that

*λ*_1_ = *λ*_2_ = *λ*_3_ = −*d* < 0 or  *λ*_4_ = (*d* + *κ* + *d*_*P*_)[*ℛ*_2_ − 1] < 0 if *ℛ*_2_ < 1 or *λ*_5_ = −(*d* + *τ*_1_) < 0 or *λ*_6_ = −(*d* + *κ*_3_ + *d*_*A*_) < 0 or *λ*_7_ = −(*d* + *d*_*P*_ + *σ*_1_ + *δ*_3_) < 0 or *λ*_8_ = −(*d* + *d*_*P*_ + *σ*_2_ + *δ*_4_) < 0 or *λ*_9_ = −(*d* + *d*_*AP*_ + *σ*_3_) < 0 or *λ*_10_ = −(*d* + *θ*) < 0 or *a*_2_*λ*^2^ + *a*_1_*λ* + *a*_0_ = 0 for *a*_2_ = 1, *a*_1_ = (*d* + *κ*_2_ + *δ*_2_) + (*d* + *κ*_1_ + *δ*_1_)[1 − (*Y*_1_^0^/*N*^0^)*ℛ*_*Y*_4__] > 0 if *ℛ*_*Y*_4__ < 1 and *a*_0_ = (*d* + *κ*_2_ + *δ*_2_)(*d* + *κ*_1_ + *δ*_1_)[1 − (*Y*_1_^0^/*N*^0^)*ℛ*_*Y*_5__) > 0 if *ℛ*_*Y*_5__ < 1.

Then, by applying Routh-Hurwitz stability criteria since *a*_2_ = 1 > 0, *a*_1_ > 0, and *a*_0_ > 0, all the eigenvalues of the Jacobian matrix are negative if *ℛ*_1_ < 1 and *ℛ*_2_ < 1, i.e., *ℛ*_3_ = max{*ℛ*_1_, *ℛ*_2_} < 1. Thus, the disease-free equilibrium point (DFE) of HIV/AIDS-pneumonia coinfection model (4) is locally asymptotically stable if

(27) $$\begin{array}{c} R_{3}=\max\left\{R_{1},R_{2}\right\}<1. \end{array}$$

☐

#### 3.3.4. Existence of Endemic Equilibrium Point (EEP) for the Full Model

The endemic equilibrium point (EEP) of full model (4) is denoted by *E*_3_^∗^ = (*Y*_1_^∗^, *Y*_2_^∗^, *Y*_3_^∗^, *Y*_4_^∗^, *Y*_5_^∗^, *Y*_6_^∗^, *Y*_7_^∗^, *Y*_8_^∗^, *Y*_9_^∗^, *Y*_10_^∗^, *Y*_11_^∗^, *Y*_12_^∗^) which occurs when the disease persists in the community. From the analysis of HIV/AIDS-only submodel (8) and the pneumonia-only submodel from (9), we have shown that there is no endemic equilibrium point if *ℛ*_1_ < 1 and there is/are an endemic equilibrium point(s) if *ℛ*_2_ < 1 implies that there is/are endemic equilibrium point(s) if *ℛ*_3_ < 1 for the coinfection model and hence there is a bifurcation point for the full model. The endemic equilibrium of system (4) is obtained as

(28) $$\begin{array}{c} \begin{array}{c} \begin{array}{c} Y_{1}^{*}=\frac{\left(1-\pi \right)\Lambda +\tau_{1}Y_{2}^{*}+\theta Y_{10}^{*}}{d+\lambda_{HC}^{*}+\lambda_{PC}^{*}},Y_{2}^{*}=\frac{\pi \Lambda }{\epsilon \lambda_{PC}^{*}+\left(d+\tau_{1}+\lambda_{HC}^{*}\right)},Y_{3}^{*}=\frac{\epsilon \lambda_{PC}^{*}Y_{2}^{*}+\lambda_{PC}^{*}Y_{1}^{*}}{\nu \lambda_{HC}^{*}+d+\kappa +d_{P}},\\ Y_{4}^{*}=\frac{\lambda_{HC}^{*}Y_{1}^{*}}{d+\kappa_{1}+\delta_{1}+\psi_{1}\lambda_{PC}^{*}},Y_{5}^{*}=\frac{\delta_{1}H_{1}^{*}}{d+\kappa_{2}+\kappa_{2}+\psi_{2}\lambda_{PC}^{*}},Y_{6}^{*}=\frac{\;\delta_{2}Y_{5}^{*}}{d+\kappa_{3}+d_{A}+\delta_{3}\lambda_{PC}^{*}}, \end{array}\\ Y_{7}^{*}=\frac{\psi_{1}\lambda_{PC}^{*}Y_{4}^{*}+\nu \lambda_{HC}^{*}Y_{3}^{*}}{d+d_{P}+\sigma_{1}+\delta_{3}},Y_{8}^{*}=\frac{\delta_{2}\lambda_{PC}^{*}Y_{5}^{*}+\delta_{3}Y_{7}^{*}}{d+d_{P}+\sigma_{2}+\delta_{4}},Y_{9}^{*}=\frac{\;\psi_{3}\lambda_{PC}^{*}Y_{6}^{*}+\delta_{4}Y_{8}^{*}}{d+d_{AP}+\kappa_{3}},\\ Y_{10}^{*}=\frac{\kappa Y_{3}^{*}}{d+\theta },Y_{11}^{*}=\frac{\kappa_{1}Y_{4}^{*}+\kappa_{2}Y_{5}^{*}+\kappa_{3}Y_{6}^{*}}{d},\text{and }Y_{12}^{*}=\frac{\kappa_{1}Y_{7}^{*}+\kappa_{2}Y_{8}^{*}+\kappa_{3}Y_{9}^{*}}{d}. \end{array} \end{array}$$

Summary of endemic equilibrium points: the explicit computation of the endemic equilibrium of coinfection model (4) given in (28) in terms of model parameters is difficult analytically; however, model (4) endemic equilibriums correspond to the following:

1. *E*_4_^∗^ = (*Y*_1_^∗^, 0, *Y*_4_^∗^, *Y*_5_^∗^, *Y*_6_^∗^, 0, 0, 0, 0, 0, *Y*_11_^∗^, 0), if *ℛ*_1_ > 1 is the pneumonia free (HIV) endemic equilibrium point. The analysis of the equilibrium *E*_1_^∗^ is similar to the endemic equilibrium *E*_1_^∗^ in model (7)
2. *E*_5_^∗^ = (*Y*_1_^∗^, *Y*_2_^∗^, *Y*_3_^∗^, 0, 0, 0, 0, 0, 0, *Y*_10_^∗^, 0, 0), if *ℛ*_2_ > 1 is the HIV/AIDS free (pneumonia) endemic equilibrium point. The analysis of the equilibrium *E*_5_^∗^ is similar to the endemic equilibrium *E*_2_^∗^ in equation (9)
3. *E*_6_^∗^ = (*Y*_1_^∗^, *Y*_2_^∗^, *Y*_3_^∗^, *Y*_4_^∗^, *Y*_5_^∗^, *Y*_6_^∗^, *Y*_7_^∗^, *Y*_8_^∗^, *Y*_9_^∗^, *Y*_10_^∗^, *Y*_11_^∗^, *Y*_12_^∗^) is the HIV/AIDS-pneumonia coinfection endemic equilibrium point. It exists when each component of *E*_6_^∗^ in equation (28) is positive and summarizes the existence of the endemic equilibrium points in the following theorem

#### 3.3.5. Bifurcation Analysis

The threshold quantity  *ℛ*_3_ = max{*ℛ*_1_, *ℛ*_2_}  is the effective reproduction number of the system (4) where *ℛ*_1_ and *ℛ*_2_ are defined as above.

**Theorem 7 .**

Model (4) exhibits the phenomenon of backward bifurcation at *ℛ*_3_ = 1 whenever the inequality *G*_1_ > *G*_2_ holds.

The phenomenon of backward bifurcation can be proved with the concept of the center manifold theory [10, 27] on coepidemic model (4). To apply this theory, the following simplification and change of variables are made.

Let *Y*_1_ = *x*_1_, *Y*_2_ = *x*_2_, *Y*_3_ = *x*_3_, *Y*_4_ = *x*_4_, *Y*_5_ = *x*_5_, *Y*_6_ = *x*_6_, *Y*_7_ = *x*_7_, *Y*_8_ = *x*_8_, *Y*_9_ = *x*_9_, *Y*_10_ = *x*_10_, *Y*_11_ = *x*_11_, and *Y*_12_ = *x*_12_ so that *N* = *x*_1_ + *x*_2_ + *x*_3_ + *x*_4_+*x*_5_,+*x*_6_+*x*_7_,+*x*_8_+*x*_9_+*x*_10_+*x*_11_+*x*_12_.

Further, by using vector notation  *X* = (*x*_1_, *x*_2_, *x*_3_, *x*_4_, *x*_5_, *x*_6_, *x*_7_, *x*_8_, *x*_9_, *x*_10_, *x*_11_, *x*_12_)^*T*^, complete model (4) can be written in the form *dX*/*dt* = *F*(*X*) with *F* = (*f*_1_, *f*_2_, *f*_3_, *f*_4_, *f*_5_, *f*_6_, *f*_7_, *f*_8_, *f*_9_, *f*_10_, *f*_11_, *f*_12_)^*T*^, as follows:

(29) $$\begin{array}{c} \begin{array}{c} \begin{array}{c} \begin{array}{c} \begin{array}{c} \begin{array}{c} \begin{array}{c} \frac{{dx}_{1}}{dt}=f_{1}=\left(1-\pi \right)\Lambda +\tau_{1}x_{2}+\theta x_{10}-\left(d+\lambda_{HC}+\lambda_{PC}\right)x_{1},\\ \frac{{dx}_{2}}{dt}=f_{2}=\pi \Lambda -\epsilon \lambda_{PC}x_{2}-\left(d+\tau_{1}+\lambda_{HC}\right)x_{2}, \end{array}\\ \frac{{dx}_{3}}{dt}=f_{3}=\epsilon \lambda_{PC}x_{2}+\lambda_{PC}x_{1}-\left(\nu \lambda_{HC}+d+\kappa +d_{P}\right)x_{3},\\ \frac{{dx}_{4}}{dt}=f_{4}=\lambda_{HC}x_{1}-\left(d+\kappa_{1}+\delta_{1}+\psi \lambda_{PC}\right)x_{4}, \end{array}\\ \frac{{dx}_{5}}{dt}=f_{5}=\delta_{1}x_{4}-\left(d+\kappa_{2}+\kappa_{2}+\psi_{2}\lambda_{PC}\right)x_{5},\\ \frac{{dx}_{6}}{dt}=f_{6}=\delta_{2}x_{5}-\left(d+\kappa_{3}+d_{A}+\psi_{3}\lambda_{PC}\right)x_{6}, \end{array}\\ \frac{{dx}_{7}}{dt}=f_{7}=\psi_{1}\lambda_{PC}x_{4}+\nu \lambda_{HC}x_{3}-\left(d+d_{P}+\sigma_{1}+\delta_{3}\right)x_{7},\\ \;\frac{{dx}_{8}}{dt}=f_{8}=\psi_{2}\lambda_{PC}x_{5}+\delta_{3}x_{7}-\left(d+d_{P}+\sigma_{2}+\delta_{4}\right)x_{8}, \end{array}\\ \frac{{dx}_{9}}{dt}=f_{9}=\psi_{3}\lambda_{PC}x_{6}+\delta_{4}x_{8}-\left(d+d_{AP}+\kappa_{3}\right)x_{9},\\ \frac{{dx}_{10}}{dt}=f_{10}=\kappa x_{3}-\left(d+\theta \right)x_{10}, \end{array}\\ \frac{{dx}_{11}}{dt}=f_{11}=\kappa_{1}x_{4}+\kappa_{2}x_{5}+\kappa_{3}x_{6}-dx_{11},\\ \frac{{dx}_{12}}{dt}=f_{12}=\kappa_{1}x_{7}+\kappa_{2}x_{8}+\kappa_{3}x_{9}-dx_{12}, \end{array} \end{array}$$

with *λ*_*HC*_ = *β*_1_/*N*[*x*_4_ + *ρ*_1_*x*_5_ + *ρ*_2_*x*_7_ + *ρ*_2_*x*_8_] where *ρ*_3_ ≥ *ρ*_2_ ≥ *ρ*_1_ ≥ 1 and *λ*_*PC*_ = *β*_2_[*x*_3_ + *ω*_1_*x*_7_ + *ω*_2_*x*_8_ + *ω*_3_*x*_9_]  where *ω*_3_ ≥ *ω*_2_ ≥ *ω*_1_ ≥ 1; then, the method entails evaluating the Jacobian of system (29) at the DFE *E*_3_^0^, denoted by *J*(*E*_3_^0^), and this gives us

(30) $$\begin{array}{c} J\left(E_{3}^{0}\right)=\left(\begin{array}{cccccccccccc} -d & \;\tau_{1} & \;F_{1} & F_{2} & F_{3} & 0 & F_{4} & F_{5} & F_{6} & \theta & 0 & 0\\ 0 & \;F_{7} & F_{8} & F_{9} & F_{10} & 0 & F_{11} & F_{12} & F_{13} & 0 & 0 & 0\\ 0 & 0 & F_{14} & 0 & 0 & 0 & F_{15} & F_{16} & F_{17} & 0 & 0 & 0\\ 0 & 0 & 0 & F_{18} & F_{19} & 0 & F_{20} & F_{21} & 0 & 0 & 0 & 0\\ 0 & 0 & 0 & \delta_{1} & F_{22} & 0 & 0 & 0 & 0 & 0 & 0 & 0\\ 0 & 0 & 0 & 0 & \delta_{2} & F_{23} & 0 & 0 & 0 & 0 & 0 & 0\\ 0 & 0 & 0 & 0 & 0 & 0 & F_{24} & 0 & 0 & 0 & 0 & 0\\ 0 & 0 & 0 & 0 & 0 & 0 & \delta_{3} & F_{25} & 0 & 0 & 0 & 0\\ 0 & 0 & 0 & 0 & 0 & 0 & 0 & d_{4} & F_{26} & 0 & 0 & 0\\ 0 & 0 & \kappa & 0 & 0 & 0 & 0 & 0 & 0 & F_{27} & 0 & 0\\ \;0 & 0 & 0 & \kappa_{1} & \kappa_{2} & \kappa_{3} & 0 & 0 & 0 & 0 & -d & 0\\ 0 & 0 & 0 & 0 & 0 & 0 & \kappa_{1} & \kappa_{2} & \kappa_{3} & 0 & 0 & -d \end{array}\right), \end{array}$$

where *F*_1_ = −*β*_2_*Y*_1_^0^, *F*_2_ = −*β*_1_(*Y*_1_^0^/(*Y*_1_^0^ + *Y*_2_^0^)), *F*_3_ = −*β*_1_*ρ*_1_(*Y*_1_^0^/(*Y*_1_^0^ + *Y*_2_^0^)), *F*_4_ = −*β*_1_*ρ*_2_(*Y*_1_^0^/(*Y*_1_^0^ + *Y*_2_^0^)) − *β*_2_*ω*_1_*Y*_1_^0^, *F*_5_ = −*β*_1_*ρ*_3_(*Y*_1_^0^/(*Y*_1_^0^ + *Y*_2_^0^)) − *β*_2_*ω*_2_*Y*_1_^0^, *F*_6_ = −*β*_2_*ω*_3_*Y*_1_^0^,  *F*_7_ = −(*d* + *τ*_1_), *F*_8_ = −*ϵβ*_2_*Y*_2_^0^, *F*_9_ = −*β*_1_(*Y*_2_^0^/(*Y*_1_^0^ + *Y*_2_^0^)), *F*_10_ = −*β*_1_*ρ*_1_(*Y*_2_^0^/(*Y*_1_^0^ + *Y*_2_^0^)),

*F*_11_ = −*ϵβ*_2_*ω*_1_*V*_*P*_^0^ − *β*_1_*ρ*_2_(*Y*_*P*_^0^/(*Y*_1_^0^ + *Y*_*P*_^0^)), *F*_12_ = −*ϵβ*_2_*ω*_2_*V*_*P*_^0^ − *β*_1_*ρ*_3_(*Y*_2_^0^/(*Y*_1_^0^ + *Y*_2_^0^)), *F*_13_ = −*ϵβ*_2_*ω*_3_*Y*_2_^0^, *F*_14_ = *ϵβ*_2_*Y*_2_^0^ + *β*_2_*Y*_1_^0^ − (*d* + *κ* + *d*_*P*_), *F*_15_ = *ϵβ*_2_*ω*_1_*Y*_2_^0^ + *β*_2_*ω*_1_*Y*_1_^0^, *F*_16_ = *ϵβ*_2_*ω*_2_*Y*_2_^0^ + *β*_2_*ω*_2_*Y*_1_^0^, *F*_17_ = *ϵβ*_2_*ω*_3_*Y*_2_^0^ + *β*_2_*ω*_3_*Y*_1_^0^, *F*_18_ = *β*_1_(*Y*_1_^0^/(*Y*_1_^0^ + *Y*_2_^0^)) − (*d* + *κ*_1_ + *δ*_1_), *F*_19_ = *β*_1_*ρ*_1_(*Y*_1_^0^/(*Y*_1_^0^ + *Y*_2_^0^)), *F*_20_ = *β*_1_*ρ*_2_(*Y*_1_^0^/(*Y*_1_^0^ + *Y*_2_^0^)), *F*_21_ = *β*_1_*ρ*_3_(*Y*_1_^0^/(*Y*_1_^0^ + *Y*_2_^0^)), *F*_22_ = −(*d* + *κ*_2_ + *δ*_2_), *F*_23_ = −(*d* + *κ*_3_ + *d*_*A*_), *F*_24_ = −(*d* + *d*_*P*_ + *σ*_1_ + *δ*_3_), *F*_25_ = −(*d* + *d*_*P*_ + *σ*_2_ + *δ*_4_), *F*_26_ = −(*d* + *d*_*AP*_ + *σ*_3_), and  *F*_27_ = −(*d* + *θ*).

Without loss of generality, consider the case when *ℛ*_2_ > *ℛ*_1_, and *ℛ*_3_ = 1, so that *ℛ*_2_ = 1. Furthermore, let *β*_2_ = *β*^∗^ is chosen as a bifurcation parameter. Solving for *β*_2_ from *ℛ*_2_ = 1 as *ℛ*_2_ = *β*_2_*ϵΛπd* + *β*_2_*Λ*(*d* + *τ*_1_) − *β*_2_*Λπd*/*d*(*d* + *τ*_1_)(*d* + *κ* + *d*_*P*_) = 1, we have got the value *β*^∗^ = *β*_2_ = *d*(*d* + *τ*_1_)(*d* + *κ* + *d*_*P*_)/*ϵΛπd* + *Λ*(*d* + *τ*_1_) − *Λπd*.

After solving the Jacobian *J*(*E*_3_^0^) of the system (29) at the DFE, with *β*_2_ = *β*^∗^, we obtained the eigenvalues as *λ*_1_ = −*d* < 0 or *λ*_2_ = −(*d* + *τ*_1_) < 0 or *λ*_3_ = 0  or *λ*_4_ = −*d* < 0 or *λ*_5_ = −*d* < 0 or *λ*_6_ = −(*d* + *θ*) < 0 or *λ*_7_ = −(*d* + *d*_*AP*_ + *κ*_3_) < 0 or *λ*_8_ = −(*d* + *κ*_3_ + *d*_*A*_) < 0 or *λ*_9_ = −(*d* + *d*_*P*_ + *σ*_1_ + *δ*_3_) < 0 or *λ*_10_ = −(*d* + *d*_*P*_ + *σ*_1_ + *δ*_4_) < 0 or

(31) $$\begin{array}{c} a_{2}\lambda^{2}+a_{1}\lambda +a_{0}=0, \end{array}$$

where *a*_2_ = 1 > 0, *a*_1_ = (*d* + *κ*_1_ + *δ*_1_)[1 − (*Y*_1_^0^/(*Y*_1_^0^ + *Y*_4_^0^))*ℛ*_*Y*_4__] + (*d* + *κ*_2_ + *δ*_2_) > 0 if *ℛ*_*Y*_4__ < 1, and *a*_0_ = *a*_0_ = (*d* + *κ*_1_ + *δ*_1_)(*d* + *κ*_2_ + *δ*_2_)[1 − (*Y*_1_^0^/(*Y*_1_^0^ + *Y*_2_^0^))*ℛ*_1_] > 0 if *ℛ*_1_ < 1.

Equation (31) has/have no positive root/s whenever *ℛ*_1_ < 1, and hence, both eigenvalues are negative. It follows that the Jacobian *J*(*E*_3_^0^) of (29) at the DFE, with *β*_2_ = *β*^∗^, denoted by *J*_*β*^∗^_, has a simple zero eigenvalue (with all other eigenvalues having negative real part). Hence, the center manifold theory [27] can be used to analyze the dynamics of model (4). In particular, the Castillo-Chavez and Song theorem [28] will be used to show that model (4) undergoes backward bifurcation at *ℛ*_*P*_ = 1.

Eigenvectors of *J*_*β*^∗^_: for the case when *ℛ*_*P*_ = 1, the right eigenvectors of the Jacobian of (29) at *β*_2_ = *β*^∗^ (denoted by *J*_*β*^∗^_) associated with the zero eigenvalue given by *u* = (*u*_1_, *u*_2_, *u*_3_, *u*_4_, *u*_5_, *u*_6_, *u*_7_, *u*_8_, *u*_9_, *u*_10_, *u*_11_, *u*_12_)^*T*^ are *u*_1_ = ((−*τ*_1_*F*_8_*F*_27_ + *F*_1_*F*_7_*F*_27_ − *θγF*_7_)/*dF*_7_*F*_27_)*u*_3_, *u*_2_ = −(*F*_8_/*F*_7_)*u*_3_, *u*_3_ = *u*_3_ > 0, *u*_10_ = (−*κ*/*F*_27_)*u*_3_ , and *u*_4_ = *u*_5_ = *u*_6_ = *u*_7_ = *u*_8_ = *u*_9_ = *u*_11_ = *u*_12_ = 0.

The left eigenvectors associated with the zero eigenvalue at *β*_2_ = *β*_2_^∗^ satisfying *v*.*w* = 1 given by *v* = (*v*_1_, *v*_2_, *v*_3_, *v*_4_, *v*_5_, *v*_6_, *v*_7_, *v*_8_, *v*_9_, *v*_10_, *v*_11_, *v*_12_) are *v*_1_ = *v*_2_ = *v*_4_ = *v*_5_ = *v*_6_ = *v*_10_ = *v*_11_ = *v*_12_=0, *v*_3_ = *v*_3_ > 0, *v*_7_ = ((−*δ*_3_*δ*_4_*F*_17_ + *δ*_3_*F*_16_*F*_26_ − *F*_15_*F*_25_*F*_26_)/*F*_24_*F*_25_*F*_26_)*v*_3_, *v*_8_ = (*δ*_4_*F*_17_ − *F*_16_*F*_26_)/*F*_25_*F*_26_*v*_3_, and *v*_9_ = −(*F*_17_/*F*_26_)*v*_3_.

After going through detailed computations and simplification, we have the following bifurcation coefficients *a* and *b* as

(32) $$\begin{array}{c} a=2v_{3}u_{1}u_{3}\frac{\partial^{2}f_{3}\left(0,0\right)}{\partial x_{1}\partial x_{3}}+2v_{3}u_{2}u_{3}\frac{\partial^{2}f_{3}\left(0,0\right)}{\partial x_{2}\partial x_{3}}=2\beta_{2}^{*}v_{3}u_{3}\left[u_{1}+\epsilon u_{2}\right]. \end{array}$$

⟹a = 2*β*_2_^∗^*v*_3_*u*_3_^2^[*G*_1_ − *G*_2_] where *G*_1_=*θκ*/*d*(*d* + *θ*) and *G*_2_ = *ϵβ*^∗^*τ*_1_*V*_*P*_^0^ + *β*^∗^(*d* + *τ*_1_)*Y*_1_^0^ + *ϵβ*^∗^*dY*_2_^0^/*d*(*d* + *τ*_1_). Thus, the bifurcation coefficient *a* is positive whenever *G*_1_ > *G*_2_. Furthermore, *b* = *v*_3_*u*_3_(*∂*^2^*f*_2_(0, 0)/*∂x*_3_*∂β*_2_) = *v*_3_*u*_3_(*ϵY*_2_^0^ + *Y*_1_^0^) > 0.

Hence, it follows from in Castillo-Chavez and Song [28] that model (4) exhibits a backward bifurcation at *ℛ*_3_ = *ℛ*_2_ = 1 whenever *G*_1_ > *G*_2_.

**Theorem 8 .**

- Model (4) will undergo backward bifurcation if *a* = *G*_1_ > *G*_2_ > 0
- Model (4) will undergo forward bifurcation if *a* = *G*_1_ > *G*_2_ < 0

## 4. Sensitivity and Numerical Analysis

### 4.1. Sensitivity Analysis

Definition. The normalized forward sensitivity index of a variable *ℛ*_3_ that depends differentiably on a parameter *p* is defined as SI(*p*) = (*∂ℛ*_3_/*∂p*)∗(*p*/*ℛ*_3_) [18].

Sensitivity indices allow us to examine the relative importance of different parameters in pneumonia and HIV/AIDS spread and prevalence. The most sensitive parameter has the magnitude of the sensitivity index larger than that of all other parameters. We can calculate the sensitivity index in terms of *ℛ*_1_ and *ℛ*_2_ since *ℛ*_3_ = max{*ℛ*_1_, *ℛ*_2_}. Sensitivity analysis results and the numerical simulation are given in this section with parameters values given in Table 3 where *N*^0^ is the total number of the initial population of complete model (4).

Using the values of parameters in Table 3, the sensitivity indices are calculated in Tables 4 and 5.

In this paper, with parameter values in Table 3, we have got *ℛ*_1_ = 1.386 at *β*_1_ = 2 implies HIV/AIDS spreads in the community and also we have got the indices as shown in Table 4. Here, sensitivity analysis shows that the human recruitment rate *Λ* and HIV/AIDS spreading rate *β*_1_ have the highest impact on the basic reproduction number of HIV/AIDS (*ℛ*_1_).

Similarly, with parameter values in Table 3, we have got *ℛ*_2_ = 9.69 at *β*_2_ = 0.2 imply that pneumonia spreads throughout the community and also we have got the indices as shown in Table 4. Here, sensitivity analysis shows that the foremost sensitive positive parameters are the human recruitment rate *Λ* and the pneumonia spreading rate *β*_2_. The foremost sensitive negative parameter is treatment rate of pneumonia (*κ*) which is inversely related to the effective reproduction number *ℛ*_2_, i.e., a smaller amount of increase in this parameter value will lead to a greater amount of reduction in the effective reproduction number while a smaller amount of decrement will cause a big increment in the basic reproduction number. Epidemiologically, the most sensitive parameters to *ℛ*_1_ and *ℛ*_2_ which can be controlled through interventions and preventions are found to be *β*_1_ and *β*_2_, respectively.

### 4.2. Numerical Analysis

In this section, numerical simulation is performed for complete HIV/AIDS-pneumonia coepidemic model (4). With ode45, we have checked the effect of some parameters in the spreading as well as for the control of pneumonia only, HIV/AIDS only, and coepidemic of HIV/AIDS and pneumonia. The parameter values put forward in Table 3 are used for numerical simulation. In the numerical simulation part, we investigated the stability of the endemic equilibrium point of complete model (4), parameter effects on the reproduction numbers, and the impact of treatment mainly on dually infected individuals in the community.

#### 4.2.1. Local Stability of Endemic Equilibrium Point of Complete Model (4)

Figure 2 shows that in the long run (after 50 years), the solutions of dynamical system (4) will be converging to its endemic equilibrium point, i.e., the endemic equilibrium point is locally asymptotically stable whenever

(33) $$\begin{array}{c} \;R_{3}=\max\left\{R_{1},R_{2}\right\}=\max\left\{1.386,9.69\right\}=9.69>1. \end{array}$$

#### 4.2.2. Effect of Parameters on the Threshold Parameter *ℛ*_2_

In this subsection, as we see in Figure 3, we have investigated the effect of pneumonia vaccination portion *π* on the pneumonia effective reproduction number  *ℛ*_2_. The figure reflects that when the value of *π* increases, the pneumonia effective reproduction number is going down, and whenever the value of *π* > 0.64 imply *ℛ*_2_ < 1. Therefore, public policymakers must concentrate on maximizing the values of pneumonia vaccination portion *π* to prevent and control pneumonia spreading.

In this subsection, as we see in Figure 4, we have investigated the effect of pneumonia spreading rate *β*_2_ on the pneumonia effective reproduction number *ℛ*_2_ by keeping the other rates as in Table 3. Figure 4 reflects that when the value of *β*_2_ increases, the pneumonia effective reproduction number *ℛ*_2_ increases, and whenever the value of *β*_2_ < 0.022 implies *ℛ*_2_ < 1. Therefore, public policymakers must concentrate on minimizing the values of pneumonia spreading rate *β*_2_ to minimize pneumonia effective reproduction number *ℛ*_2_.

#### 4.2.3. Effect of Pneumonia Treatment Rate on Infectious Population

In this subsection, as we see in Figure 5, we have investigated the effect of *κ* in decreasing the number of pneumonia-only infectious populations. The figure reflects that when the values of *κ* increase, the number of pneumonia-only infectious population is going down. Therefore, public policymakers must concentrate on maximizing the values of treatment rate *κ* to pneumonia disease.

#### 4.2.4. Effect of Treatment Rates on HIV/AIDS Infectious Population

In this subsection, as we see in Figures 6–8, respectively, we have investigated the effects of *κ*_1_, *κ*_2_, and *κ*_3_ in decreasing the number of acute HIV only, chronic HIV only, and AIDS-infected population, respectively. The figures reflect that when the values of *κ*_1_, *κ*_2_, and *κ*_3_ increase, the number of acute HIV only, chronic HIV only, and AIDS-infected population is going down, respectively. Therefore, public policymakers must concentrate on maximizing the values of treatment rate of individuals to HIV/AIDS infection.

#### 4.2.5. Effect of HIV/AIDS Transmission Rate on Coinfectious Population

In this section, we see in Figure 9 the effect of the spreading rate of HIV/AIDS *β*_1_ on the acute HIV-pneumonia coepidemic population *Y*_7_. The figure reflects that as the value of the transmission rate (*β*_1_) of HIV/AIDS is increased, the coepidemic population increases, which means the expansion of coepidemic of HIV/AIDS-pneumonia will increase. To control coepidemic of HIV/AIDS-pneumonia, decreasing the spreading rate of HIV/AIDS is important. Therefore, stakeholders must concentrate on decreasing the spreading rate of HIV/AIDS by using the treatment and appropriate method of prevention mechanism to bring down the expansion of coepidemic in the community.

#### 4.2.6. Effect of Treatment Rates on HIV/AIDS-Pneumonia Coepidemic Population

In this subsection, as we see in Figures 10–12, we have investigated the effects of treatment rates *σ*_1_, *σ*_2_, and *σ*_3_ in decreasing the number of acute HIV and pneumonia, chronic HIV and pneumonia, and AIDS and pneumonia coinfectious population, respectively. The figures reflect that when the values of *σ*_1_, *σ*_2_, and *σ*_3_ increase, the number of acute HIV-pneumonia, chronic HIV-pneumonia, and AIDS-pneumonia coepidemic population is going down, respectively. Therefore, public policymakers must concentrate on maximizing the values of treatment rates of HIV/AIDS-pneumonia coepidemic population.

## 5. Discussion

In Section 1, we reviewed and introduced the epidemiology of HIV/AIDS, pneumonia, and HIV/AIDS-pneumonia coepidemic. In Section 2, we construct the compartmental HIV/AIDS-pneumonia coepidemic dynamical system using an ordinary differential equation and we partitioned it into twelve distinct compartments. In Section 3, we analyzed the model qualitatively. To study the qualitative behavior of complete model (4), first, we split the complete model into two, which are HIV/AIDS-only and pneumonia-only models. The qualitative behaviors, i.e., the positivity of future solutions of the models, boundedness of the dynamical system, disease-free equilibrium points, basic reproduction numbers, endemic equilibriums, stability analysis of disease-free equilibrium points, stability analysis of endemic equilibrium points, bifurcations analysis of pneumonia-only model and the complete HIV/AIDS-pneumonia coepidemic model, and sensitivity analysis of reproduction numbers of HIV/AIDS-only and pneumonia-only model, are analyzed in their respective order, and numerically, we experimented on the stability of endemic equilibrium point of the HIV/AIDS-pneumonia coepidemic model, effect of basic parameters in the expansion or control of pneumonia only, HIV/AIDS only, and HIV/AIDS-pneumonia coepidemic infections and parameter effects on the infected population. From the result, we conclude that increasing both the pneumonia treatment rate and pneumonia vaccination portion rate has a great contribution to bringing down pneumonia infection as well as the coepidemic in the community. Similarly, increasing the HIV/AIDS treatment rates also has a contribution to minimizing the expansion of HIV/AIDS infection. The coepidemic treatment rates also influence minimizing coepidemic population if its value is increased. The other result obtained in this section is that decreasing the transmission rates has a great influence of controlling coepidemic in the population.

## 6. Conclusion

A realistic compartmental mathematical model on the spread and control of HIV/AIDS-pneumonia coepidemic incorporating pneumonia vaccination and treatment for both infections are available at each stage of the infection in a population constructed and analyzed. We have shown the positivity and boundedness of the complete HIV/AIDS-pneumonia coepidemic model. Using center manifold theory, we have shown that the pneumonia-only infection and the complete HIV/AIDS-pneumonia coepidemic models undergo the phenomenon of backward bifurcation whenever their corresponding effective reproduction numbers are less than one. The complete model has a disease-free equilibrium that is locally asymptotically stable whenever the maximum of the reproduction numbers of the two submodels described above is less than one. Numerical simulation shows that the complete HIV/AIDS-pneumonia coepidemic model endemic equilibrium point is locally asymptotically stable when its effective reproduction number is greater than one. These results have important public health implications, as they govern the elimination and/or persistence of the two diseases in a community. By analyzing the various associated reproduction numbers, we have shown that the impact of some parameters changes on the associated reproduction numbers to give future recommendations for the stakeholders in the community. From the numerical result, we have got the complete model reproduction number is *ℛ*_3_ = max{*ℛ*_1_, *ℛ*_2_} = max{1.386, 9.69 } = 9.69  at *β*_1_ = 2 and *β*_2_ = 0.2. From our numerical result, we recommend that public policymakers must concentrate on maximizing the values of pneumonia vaccination portion and treatment rate of individuals to pneumonia disease. Finally, some of the main epidemiological findings of this study include pneumonia vaccination and treatment against disease has the effect of decreasing the pneumonia and coepidemic disease expansion and prevalence and reducing the progression rate of HIV infection to the AIDS stage and the HIV/AIDS prevalence.

### 6.1. Limitation of the Study

Due to conflict in our country Ethiopia, it is difficult to incorporate experimental data in the study.

## Figures and Tables

**Figure 1:** Flowchart of the HIV/AIDS-pneumonia coinfection model (4) where *λ*_*HC*_ and *λ*_*PC*_ are given in (2) and (3), respectively.

**Figure 2:** Local stability of endemic equilibrium point of the coepidemic model (4) whenever *ℛ*_1_ = 1.386 at *β*_1_ = 2 and *ℛ*_2_ = 9.69 at *β*_2_ = 0.2.

**Figure 3:** Effect of pneumonia vaccination on *ℛ*_2_.

**Figure 4:** Effect of pneumonia transmission on *ℛ*_2_.

**Figure 5:** Effect of treatment on pneumonia-infected population.

**Figure 6:** Effect of treatment on acute HIV-infected population at *β*_1_ = 0.5.

**Figure 7:** Effect of treatment on chronic HIV-infected population at *β*_1_ = 0.5.

**Figure 8:** Effect of treatment on AIDS patients at *β*_1_ = 0.5.

**Figure 9:** Effect of *β*_1_ on acute HIV-pneumonia coepidemic population.

**Figure 10:** Effect of treatment on acute HIV and pneumonia coepidemic.

**Figure 11:** Effect of treatment on chronic HIV and pneumonia.

**Figure 12:** Effect of treatment on AIDS and pneumonia coepidemic.

**Table 1:** Descriptions of model parameters.

Parameter	Interpretations
*d*	Natural mortality rate
*Λ*	Human recruitment rate
*δ*_1_	Development rate from acute HIV to chronic HIV infection
*δ*_2_	Development rate from chronic HIV to AIDS stage
*ϵ*	The proportion of the serotype not covered by the vaccine
*θ*	Immunity loss rate
*ψ*_1_	Alteration rate indicating acute HIV infection is more vulnerable to pneumonia
*ψ*_2_	Alteration rate indicating chronic HIV infection is more vulnerable to pneumonia
*ψ*_3_	Alteration rate indicating AIDS patient is more vulnerable to pneumonia
*λ*_*HC*_	HIV/AIDS standard incidence rate
*λ*_*PC*_	Pneumonia mass action incidence rate
*δ*_3_	Development rate from acute HIV-pneumonia to chronic HIV-pneumonia coepidemics
*δ*_4_	Development rate from chronic HIV-pneumonia to AIDS-pneumonia coepidemics
*d*_*P*_	Pneumonia death rate
*d*_*A*_	AIDS death rate
*d*_*AP*_	AIDS-pneumonia death rate
*κ*	Pneumonia infection treatment rate
*κ*_1_	Acute HIV infection treatment rate
*τ*_1_	Vaccination waning rate
*κ*_2_	Chronic HIV infection treatment rate
*κ*_3_	AIDS patients treatment rate
*σ*_1_	Acute HIV-pneumonia coepidemic treatment rate
*σ*_2_	Chronic HIV-pneumonia coepidemic treatment rate
*σ*_3_	AIDS-pneumonia coepidemic treatment rate
*β*_1_	Transmission rate of HIV
*β*_2_	Transmission rate of pneumonia

**Table 2:** Definitions of variables.

Variables	Definitions
*Y*_1_	Vulnerable to both HIV and pneumonia class
*Y*_2_	Pneumonia-vaccinated class
*Y*_3_	Pneumonia-infected class
*Y*_4_	Acute HIV-infected class
*Y*_5_	Chronic HIV-infected class
*Y*_6_	AIDS patients class
*Y*_7_	Acute HIV-pneumonia coepidemic class
*Y*_8_	Chronic HIV-pneumonia coepidemic class
*Y*_9_	AIDS-pneumonia coepidemic class
*Y*_10_	HIV/AIDS treatment class
*Y*_11_	Pneumonia treatment class
*Y*_12_	Coepidemics treatment class

**Table 3:** Parameter values used for the full HIV/AIDS-pneumonia coepidemic model simulation.

Parameter	Value	Source
*Λ*	0.0413∗*N*^0^	Estimated
d	0.02	Estimated
*δ*_1_	0.498	[7]
*δ*_2_	0.08	[7]
*δ*_3_	0.2885	[6]
*δ*_4_	0.3105	[6]
*ψ*_1_	1.1	Assumed
*ψ*_2_	1.2	Assumed
*ψ*_3_	1.4	Assumed
*ν*	1	Assumed
*d*_*P*_	0.1	[16]
*θ*	0.1	[18]
*d*_*A*_	0.333	[6]
*π*	0.2	[18]
*τ*_1_	0.0025	[18]
*ϵ*	0.002	[18]
*d*_*AP*_	0.42	Assumed
*κ*	0.2	[18]
*κ*_1_	0.2	[7]
*κ*_2_	0.15	[7]
*κ*_3_	0.13	Assumed
*σ*_1_	0.498	[7]
*σ*_2_	0.08	[7]
*σ*_3_	0.230	Assumed
*β*_1_	Variable	[6]
*β*_2_	Variable	[6]
*ρ*_1_, *ρ*_2_, *ρ*_3_, *ω*_1_, *ω*_2_, *ω*_3_	1.2,1,1,1,1,1	Assumed

**Table 4:** Sensitivity indices of *ℛ*_3_ = *ℛ*_1_.

Sensitivity index	Values
SI(*β*_1_)	+1
SI(*ρ*_1_)	+0.6134
SI(*δ*_1_)	- 0.0639
SI(*d*)	-0.3150
SI(*κ*_1_)	-0.1371
SI(*κ*_2_)	-0.0264
SI(*δ*_2_)	-0.0141

**Table 5:** Sensitivity indices of *ℛ*_3_ = *ℛ*_2_.

Sensitivity index	Values
SI(*Λ*)	+1
SI(*β*_2_)	+1
SI(*d*)	-0.4421
SI(*κ*)	-0.6559
SI(*d*_*P*_)	-0.3852
SI(*π*)	-0.3852
SI(*ϵ*)	-0.3852
SI(*τ*_1_)	-0.3852

## Data Availability

Data used to support the findings of this study are included in the article.
